This article has been retracted.

# A Deep Insight Into CAR-T Cell Therapy in Non-Hodgkin Lymphoma: Application, Opportunities, and Future Directions

**DOI:** 10.3389/fimmu.2021.681984

**Published:** 2021-06-23

**Authors:** Faroogh Marofi, Heshu Sulaiman Rahman, Muhammad Harun Achmad, Klunko Nataliya Sergeevna, Wanich Suksatan, Walid Kamal Abdelbasset, Maria Vladimirovna Mikhailova, Navid Shomali, Mahboubeh Yazdanifar, Ali Hassanzadeh, Majid Ahmadi, Roza Motavalli, Yashwant Pathak, Sepideh Izadi, Mostafa Jarahian

**Affiliations:** ^1^ Department of Hematology, Faculty of Medicine, Tabriz University of Medical Sciences, Tabriz, Iran; ^2^ Immunology Research Center, Tabriz University of Medical Sciences, Tabriz, Iran; ^3^ College of Medicine, University of Sulaimani, Sulaimaniyah, Iraq; ^4^ Department of Medical Laboratory Sciences, Komar University of Science and Technology, Sulaimaniyah, Iraq; ^5^ Department of Pediatric Dentistry, Faculty of Dentistry, Hasanuddin University, Makassar, Indonesia; ^6^ Department of Economics and Industrial Engineering, St. Petersburg University of Management and Economics, St. Petersburg, Russia; ^7^ Department of Postgraduate and Doctoral Studies, Russian New University, Moscow, Russia; ^8^ Faculty of Nursing, HRH Princess Chulabhorn College of Medical Science, Chulabhorn Royal Academy, Bangkok, Thailand; ^9^ Department of Health and Rehabilitation Sciences, College of Applied Medical Sciences, Prince Sattam bin Abdulaziz University, Al Kharj, Saudi Arabia; ^10^ Department of Physical Therapy, Kasr Al-Aini Hospital, Cairo University, Giza, Egypt; ^11^ Department of Prosthetic Dentistry, Sechenov First Moscow State Medical University, Moscow, Russia; ^12^ Stem Cell Transplantation and Regenerative Medicine, Department of Pediatrics, Stanford University School of Medicine, Palo Alto, CA, United States; ^13^ Stem Cell Research Center, Tabriz University of Medical Sciences, Tabriz, Iran; ^14^ Taneja College of Pharmacy, University of South Florida, Tampa, FL, United States; ^15^ Department of Pharmaceutical Science, Faculty of Pharmacy, Airlangga University, Subaraya, Indonesia; ^16^ German Cancer Research Center, Toxicology and Chemotherapy Unit (G401), Heidelberg, Germany

**Keywords:** chimeric antigen receptor, non-Hodgkin’s lymphoma, CD-19, target therapy, CAR T cells

## Abstract

Non-Hodgkin’s lymphoma (NHL) is a cancer that starts in the lymphatic system. In NHL, the important part of the immune system, a type of white blood cells called lymphocytes become cancerous. NHL subtypes include marginal zone lymphoma, small lymphocytic lymphoma, follicular lymphoma (FL), and lymphoplasmacytic lymphoma. The disease can emerge in either aggressive or indolent form. 5-year survival duration after diagnosis is poor among patients with aggressive/relapsing form of NHL. Therefore, it is necessary to understand the molecular mechanisms of pathogenesis involved in NHL establishment and progression. In the next step, we can develop innovative therapies for NHL based on our knowledge in signaling pathways, surface antigens, and tumor milieu of NHL. In the recent few decades, several treatment solutions of NHL mainly based on targeted/directed therapies have been evaluated. These approaches include B-cell receptor (BCR) signaling inhibitors, immunomodulatory agents, monoclonal antibodies (mAbs), epigenetic modulators, Bcl-2 inhibitors, checkpoint inhibitors, and T-cell therapy. In recent years, methods based on T cell immunotherapy have been considered as a novel promising anti-cancer strategy in the treatment of various types of cancers, and particularly in blood cancers. These methods could significantly increase the capacity of the immune system to induce durable anti-cancer responses in patients with chemotherapy-resistant lymphoma. One of the promising therapy methods involved in the triumph of immunotherapy is the chimeric antigen receptor (CAR) T cells with dramatically improved killing activity against tumor cells. The CAR-T cell-based anti-cancer therapy targeting a pan–B-cell marker, CD19 is recently approved by the US Food and Drug Administration (FDA) for the treatment of chemotherapy-resistant B-cell NHL. In this review, we will discuss the structure, molecular mechanisms, results of clinical trials, and the toxicity of CAR-T cell-based therapies. Also, we will criticize the clinical aspects, the treatment considerations, and the challenges and possible drawbacks of the application of CAR-T cells in the treatment of NHL.

## Introduction

Non-Hodgkin’s lymphoma (NHL) is the seventh common malignancy in the United States, mostly regarded as a malignancy with good prognoses and 5-year survival of approximately 70%. The most common types of NHL are diffuse large B cell lymphoma (DLBCL), follicular lymphoma (FL), and mantle cell lymphoma (MCL) (1). The typical therapeutic methods for lymphoma include radiation therapy, chemotherapy, immunotherapy, and so on. However, in approximately 20-30% of all patients with lymphoma, especially those with DLBCL (the most common invasive subtype), resistance to these treatment lines will develop (2, 3). The hematopoietic stem cell transplant (HSCT) is one of the standard care in patients with relapsed and refractory disease who have survived chemotherapy (4). However, due to underlying comorbidities and chemo-resistance disease, about 40% of patients may not be qualified for HSCT. Even about half of the patients treated with HSCT tend to relapse (5). In other words, the outcome of this treatment in patients with relapsed/refractory (R/R) disease, especially in DLBCL patients, is not entirely satisfactory. Accordingly, the presence of new therapies that improve therapeutic outcomes in patients with recurrent or refractory lymphoma is needed (6). Recently, T-cell immunotherapies with the CARs have been widely applied and have shown notable consequences in the treatment of B-cell malignancies (7). Unlike normal T cells, CAR-T cells detect unprocessed antigens. In other words, they recognize the tumor cells independently of the human leukocyte antigen (HLA) system and then eradicates them. This feature overcomes the main mechanisms of tumor escape such as defective antigen processing and decreased expression of class I HLA molecules, which prevents the recognition of HLA-restricted T cells (8, 9). The genetic sequence of the CAR molecule is transferred to T cells after loading into viral or non-viral vectors and then used to target tumor cells (10). The importance of this technology has recently been fully understood following the dramatic effect of CD19-specific CAR-T cells against the treatment-resistant B cell malignancies illustrated in primary-phase clinical trials. CD19-specific CAR-T cells have been widely used to treat B-cell lymphoma since most B-cell NHLs also highly express the CD19 marker. However, the clinical effect of anti-CD19 CAR-T cells in patients with ALL seems more significant than in patients with lymphoma. In many patients with lymphoma in whom standard care approaches have been ineffective, utilization of CARs has yielded significant responses (6). In general, unlike B-cell lymphomas, peripheral T-cell lymphomas are composed of a heterogeneous set of diseases with a poor prognosis (11). At present, due to limited antigen availability, the treatment of T cell lymphomas is very challenging and there are few T cell therapies against the antigen of T cell lymphoma (12, 13). However, recurrent relapses and resistance to the therapeutic methods lead to failure to achieve treatment in all patients (13). This study aimed to evaluate CAR-T cell products in NHL patients and to describe the unique aspects of their use for the treatment of these patients.

## Current Immunotherapeutic Approaches for NHL’s

The identification of different oncogenic signaling pathways is considered an attractive therapeutic mark in B cell malignancies. Disorder of the BCR pathway is a common feature in the pathogenesis of B-NHL. Besides, targeting BCR pathway enzymes like phosphoinositol-3 kinase (PI3K), spleen tyrosine kinase (Syk) and Bruton’s tyrosine kinase (Btk) has been largely successful in treating B-NHL subtypes. Also, inhibition of the microenvironment using immunomodulatory agents and checkpoint inhibitors, and targeting the anti-apoptotic protein of B-cell lymphoma 2 (Bcl-2), can be other attractive therapies (14) (**Table 1**).

**Table 1:** Immunotherapeutic approaches for B-Cell Non-Hodgkin’s lymphomas.

Class	Agent	Target	Histologic subtypes
**Monoclonal antibodies**	Rituximab	CD20	FL, DLBCL, and MCL
	Epratuzumab	CD22	FL, DLBCL, and
	Galiximab	CD80	B-cell lymphoma
	Tafasitamab	CD19	MCL, FL, and DLBCL
	Otlertuzumab	CD37	NHL and CLL
	MEDI-551	CD19	FL and DLBCL
**Antibody drug conjugates**	Polatuzumab Vedotin	CD79b	DLBCL
	Brentuximab Vedotin	CD30	DLBCL
	Pinatuzumab Vedotin	CD22	DLBCL and FL
	Vorsetuzumab Mafodotin	CD70	CD70-positive NHL, and metastatic renal cell carcinoma
	Inotuzumab Ozogamicin	CD22	NHL, HCL, CLL, and B-cell ALL
	Coltuximab Ravtansine	CD19	DLBCL
	IMGN529	CD37	B-NHL
**Btk inhibitors**	Ibrutinib	Btk	Marginal zone lymphoma, MCL, WM, and CLL
	Acalabrutinib	Btk	Mantle cell lymphoma and CLL
**PI3K inhibitors**	Copanlisib	PI3Kα/PI3Kδ	B-cell lymphomas, FL, and CLL
	Duvelisib	PI3K	FL and CLL/SLL
	Idelalisib	PI3Kδ	B-NHL, FL, and SLL
**Syk inhibitors**	Entospletinib	Syk	MCL, DLBCL, CLL, and AML
	Fostamatinib	Syk	Lymphoma, autoimmune thrombocytopenia, rheumatoid arthritis, IgA nephropathy, and autoimmune hemolytic anemia
**Bcl-2 inhibitors**	Navitoclax	Bcl-xL, Bcl-2, Bcl-w, and Mcl-1/A1	NHL, ALL, and CLL
	Venetoclax	Bcl-2	NHL (MCL, FL, and DLBCL)
**Checkpoint inhibitors**	Durvalumab	PD-L1	Lymphoma
	Nivolumab	PD-1	FL
	Pembrolizumab	PD-1-PD-L1/PD-L2	PMBCL
	Pidilizumab	PD-1	DLBCL

Btk, Bruton’s tyrosine kinase; PI3K, phosphatidyl-inositol-3-kinase; Syk, spleen tyrosine kinase, Bcl-2, B-cell lymphoma; NHL, Non-Hodgkin’s lymphoma; DLBCL, diffuse large B-cell lymphoma; FL, follicular lymphoma; PMBCL, mediastinal B cell lymphoma; CLL/SLL, chronic lymphocytic leukemia/small lymphocytic lymphoma; HCL, hairy cell leukemia; WM, Waldenstrom’s macroglobulinemia; AML, acute myeloid leukemia.

### Monoclonal Antibodies (mAbs)

One of the most prosperous therapeutic strategies for the treatment of NHL is utilization of mAbs. The emergence of Rituximab as an anti-CD20 antibody had a significant impact on the treatment of this group of diseases. Despite the successes, how to optimize the use, the optimal duration of treatment, and the best times to administer mAbs, especially Rituximab in the NHL have not yet been determined. It is also necessary to identify the mechanisms that develop resistance to Rituximab to increase the effectiveness of this and other similar drugs.

#### Rituximab

Rituximab [Rituxan], a chimeric anti-CD20 mAb, was the early antibody approved by the FDA for the cure of R/R low-grade NHL or FL. Approval was based on an experiment in which 166 patients with indolent NHL received Rituximab and ultimately had a complete remission (CR) rate of 6% and an overall response rate (ORR) of 48% (15). Also, Rituximab activity was used as a second-line treatment in patients with invasive DLBCL or MCL but showed relatively lower therapeutic effect (16).

#### Epratuzumab

Epratuzumab, the humanized IgG1 version of LL2 (anti-CD22 murine mAb), was designed to increase the half-life and effective performance, and reduce immunogenicity potential (17). The elementary clinical studies of this antibody labeled with ^111^In/^90^Y and ^131^I have shown evidence of tumor localization, as well as the therapeutic activity for radioimmunoconjugate (18). The exact mechanism of action of Epratuzumab has not been elucidated, but binding of human CD22 to mAbs may induce tyrosine phosphorylation of the cytoplasmic tail of CD22, binding of tyrosine phosphatase SHP-1, and ultimately inhibiting B cell receptor signaling (19).

#### Galiximab

Galiximab is a cynomolgus macaque chimeric IgG1 mAb that is designed to target CD80 and the treatment of B-cell lymphoma. This antibody is not structurally distinct from human antibodies and therefore cannot produce significant immunogenicity in humans. To date, several preclinical studies have demonstrated the antitumor activity of Galiximab alone or in combination with Rituximab against different B cell lymphoma cell lines *in-vitro*/*in-vivo* (20, 21). The mechanism of activity of Galiximab is not well understood but clinical studies with Galiximab have shown increased apoptosis and antibody-dependent cell-mediated cytotoxicity (ADCC), and decreased proliferation in various B cell lymphoma cells (22).

#### Tafasitamab

Tafasitamab (MOR208, XmAb5574) is a humanized Fc-engineered anti CD19 mAb that its preclinical activity has been shown in patients with R/R NHL including MCL, FL, and DLBCL (23). The Fc engineering, comprising the replacement of S239D and I332E amino acids is advantageous by reducing binding of FcγRIIa inhibitory receptor and increasing FcγRIIIa binding affinity on effector cells, leading to the enhancement of antigen-dependent cell-mediated phagocytosis and antigen-dependent cell-mediated cytotoxicity compared to using unmodified G1 CD19 antibodies. MOR208 potentially leads to disruption of B cell antigen receptor signaling resulting in cytotoxicity (24, 25).

#### Otlertuzumab

Otlertuzumab (TRU-016) is a protein therapeutic developed using the Modular Protein Technology (ADAPTIRTM platform) that targets the CD37 molecule. Otlertuzumab, through binding to the CD37 receptor, leads to an increase in BIM proapoptotic protein expression and apoptosis induction (26). Preclinical studies show that Otlertuzumab mediates apoptosis and FcDCC (Fc-dependent cytotoxicity) against NHL cells and chronic lymphocytic leukemia (CLL) *in vitro* and *in-vivo* (27). Besides, Otlertuzumab activity was shown to be dependent on NK cell function in several B cell malignancy xenograft models (27). Other studies have shown that blocking CD20 on the surface of target B cells with Otlertuzumab may have therapeutic benefits, especially in CLL (28, 29), because the signal resulted from Otlertuzumab is provided by interacting with CD37 separately from CD20.

#### MEDI-551

MEDI-551 is a fucosylated anti-CD19 mAb which has antitumor activity against B cell malignancies alone or in combination with Rituximab (30). In phase 1 studies, unprotected safety characteristics and single-agent activity of MEDI-551 were observed in R/R FL and DLBCL with an overall response rate of 24% (31).

### Antibody-Drug Conjugates (ADCs)

ADCs are a group of molecules made up of a mAb conjugated with a potent cytotoxic agent using a chemical linker. The linkers in these structures are cleaved by reduction, alterations in pH, or by proteases, and the drug is preferentially released at the tumor region (32). By choosing mAb against tumor-specific antigens, ADCs enable the targeted delivery of cytotoxic agents to cancer cells. In this section, the ADCs utilized to treat NHL will be discussed. ADCs change the treatment patterns of these diseases by increasing performance and improving tolerance to current chemotherapy-based regimens (33).

#### Polatuzumab Vedotin

Polatuzumab vedotin is an ADC comprised of an anti-CD79b mAb and an anti-mitotic agent called mono-methyl auristatin E (MMAE) (34). This therapeutic agent detects the CD79b protein from the B cell receptor complex and after binding to it, inhibits tubulin polymerization by entering the cytotoxic payload of MMAE drug into B-cell, leading to the death of the target cell. Targeting the CD79b pan-B marker is ideal in patients who may later need CD19-targeted CAR-T cell therapy because it will not develop resistance to CD19 regimens (35).

#### Brentuximab Vedotin

Brentoximab vedotin (BV) consists of an anti-CD30 mAb that binds to MMAE *via* a biodegradable ligand (36). After ADC binding, MMAE cleaves and undergoes endocytosis, then disrupts microtubules, arresting the cell cycle and inducing apoptosis (37). Recently, in a phase II study in DLBCL, the function of BV was investigated with an ORR of 44% (38).

#### Pinatuzumab Vedotin

Pinatuzumab Vedotin (DCDT2980S) is a humanized anti-CD22 IgG1 connected to the MMAE *via* the cathepsin-B-sensitive dipeptide (valine-citrulline, VC) linker. Binding of MMAE to microtubules arrests cell cycle in the G2/M stage and induces apoptosis (33). This ADC has been studied alone and in combination with Rituximab in CLL and NHL in phase I and II clinical trials. The results showed that (DCDT2980S) can be used as a potential therapeutic option in patients with R/R DLBCL and FL.

#### Vorsetuzumab Mafodotin

Vorsetuzumab mafodotin (SGN-75) is composed of a humanized mAb targeting CD70 (h1F6) conjugated to the monomethyl auristatin F (MMAF) *via* the noncleavable maleimidocaproyl (MC) linker (39). MMAF is stronger than MMAE but less permeable to cells (40). The lysosomal degradation of this ADC causes the generation of cysteine-MC-MMAF in cancer cells (41). SGN-75 was investigated in a phase I clinical trial for CD70-positive R/R NHL and metastatic renal cell carcinoma (RCC).

#### Inotuzumab Ozogamicin

Inotuzumab is an anti-CD22 humanized IgG4 mAb, while ozogamicin is derived from calicheamicins, a group of potent anticancer antibiotics that cause strand cleavage in the DNA minor groove, cell cycle arrest, and eventually leading to leukemic cell apoptosis (42). The CD22 receptor is a very ideal therapeutic target because in most cases of B-cell hematologic malignancies such as NHL, hairy cell leukemia, CLL, and B-cell ALL, it is expressed in tumor tissues and not seen in normal tissues such as B lymphocyte precursors and hematopoietic stem cells (43).

#### Coltuximab Ravtansine (SAR3419)

SAR3419 (huB4/DM4) is a novel Ab–drug conjugate made from a humanized IgG1 anti-CD19 mAb (huB4) bound to a potent cytotoxic agent, a maytansine-derivative chemical agent (DM4). Phase I trials based on preclinical studies have illustrated optimistic antitumor activity of this drug with admissible safety results in human B-lymphoma models (44).

#### IMGN529 (CD37 ADC)

IMGN529 is a novel ADC for the treatment of CLL and B-NHL that consists of an anti-CD37 MAb bound to maytansinoid (DM1) toxin, a potent anti-tubulin. Previously, the therapeutic effects of ^133^I-labeled CD37 MAb in the B-NHL have been investigated (45). The antitumor activity of IMGN529 has been assessed *in vitro* and xenograft models (46). Furthermore, its safety and tolerability in patients with R/R B-NHL in phase I, an open-label trial (NCT01534715) were evaluated.

### Btk Inhibitors

Disruption of the B cell receptor pathway is closely related to the spread of B cell malignancies. This has made it possible to develop component inhibitors and various important steps along this pathway. Btk is a molecule present in the early BCR signaling pathway that plays an important role in regulating various cell functions including proliferation, differentiation, and survival in this type of malignancy and has been considered as a therapeutic target in this disease (47, 48).

#### Ibrutinib

Ibrutinib, the irreversible Btk inhibitor, has been approved for the treatment of a variety of B cell malignancies (49) including marginal zone lymphoma, MCL, Waldenström macroglobulinemia (WM), and CLL. It has also been shown that Ibrutinib also suppresses Th2 cells and enhances Th1-mediated immunity by inhibiting Interleukin-2 (IL-2) inducible T-cell kinase (ITK) (50).

#### Acalabrutinib

Acalabrutinib (ACP-196) is a second-generation inhibitor of Btk with a selective kinase activity pattern that covalently binds to the cysteine-481 residue at Btk and inhibits it more strongly than Ibrutinib (51). Furthermore, Acalabrotinib has shown an acceptable outcome in early clinical trials in patients with relapsed and refractory CLL (52).

### PI3K Inhibitors

PI3K has three distinct classes (I, II, and III). The class I of PI3K pathway with 4 isoforms (α, β, γ, and δ) is most associated with the expansion and survival of malignancies and is one of the therapeutic targets of cancer (53). PI3K-α and-β are ubiquitously expressed, while the expression of PI3K-γ and -δ is more limited to leukocytes (54). Mutations and overexpression of PI3Kα are oncogenic and have been identified in various subtypes of cancer (55). Increased copy number and elevated PI3Kα protein expression have also been recognized in different lymphomas, indicating the basic role of PI3Kα in lymphomagenesis (56). Simultaneous silencing of PI3Kα and -δ is required for efficient blockage of PI3K signaling in clinical trials (57). Studies have shown that a combination of PI3Kα and δ-isoform inhibitors is required to suppress phospho-Akt and NFkB and PI3K pathways (56, 58). Therefore, molecular evaluation of PI3Kα/δ and the use of its inhibitors can be a promising therapeutic approach to eradicate lymphoma. Duvelisib, Copanlisib, and Idelalisib are three FDA-approved agents for the targeting of PI3Kδ in CLL/SLL and FL neoplastic B cells.

#### Copanlisib

Copanlisib is a PI3Kα/PI3Kδ inhibitor that has been approved as the third line of treatment for R/R FL. Besides, the antitumor activity of Copanlisib has been demonstrated in preclinical models of CLL and B-cell lymphomas (59) These researches eventually led to the first human study of Copanlisib in NHL patients.

#### Duvelisib

Duvelisib (IPI-145) is a second-generation inhibitor of PI3K that is used to treat relapsed FL and CLL/SLL after the failure of other treatments. Duvelisib also impedes the expression of PI3Kγ isoform in myeloid cells, T cells, and so on whereas Copanlisib, targets the PI3Kα isoform expressed in some types of NHL along with PI3Kδ (60). Treatment with Duvelisib by inhibiting PI3K/AKT/mTOR signaling pathway the homing and chemotaxis of CLL/SLL cells and leads to *in vitro* apoptosis (61). Thus, pharmacologic targeting of PI3Kγ reduces the migration rate of CLL/SLL cells, but the effect of Duvelisib on migration inhibition is greater than selective single isoform inhibitors (62).

#### Idelalisib

Idelalisib (CAL-101, GS-1101) is a potent inhibitor of PI3Kδ isoform and significantly suppresses B-NHL progression. The use of Idelalisib alone in patients with small lymphocytic lymphoma and FL and combination with Rituximab in patients with CLL has been approved (63).

### Syk Inhibitors

Syk is a non-receptor cytoplasmic kinase that is primarily expressed in hematopoietic cells and is one of the essential components in BCR signaling (64). Syk activation leads to BCR signal initiation through binding to adapter proteins and phosphorylation signaling mediators including Btk, B-cell linker protein (BLNK), and phospholipase Cγ2 (PLC-γ2), leading to differentiation, cell proliferation, and survival (65). Aberrant Syk signaling is involved in the pathogenesis of multiple B-cell malignancies, such as constitutive Syk activation (66) and overexpression of the protein and mRNA levels of Syk (67). As a result, Syk is an attractive target for the treatment of B-cell malignancies.

#### Entospletinib

Entospletinib (GS-9973) is a selective Syk inhibitor and its impacts were evaluated in phase 2 of the study in patients with MCL and R/R NHL (68). As a result, Entospletinib showed a toxic profile and intermediate single-agent activity in NHL, although its toxicity was controllable compared to other BCR pathway inhibitors such as Ibrutinib and Idelalisib.

#### Fostamatinib

Fostamatinib is a prodrug of the active compound R406 and a potent inhibitor of the enzyme Syk, which is administered in an oral formulation (69). So far, the clinical trials of Fostamatinib have been accomplished on autoimmune thrombocytopenia, rheumatoid arthritis, IgA nephropathy, autoimmune hemolytic anemia, and lymphoma (70, 71). The evidence from several human clinical trials has revealed that daily administration of this drug significantly reduces Syk activity without any adverse effects on hemostasis or innate immunity (69).

### Bcl-2 Inhibitors

BCL2 is a gene with unknown function that was discovered as the anonymous partner of the heavy chain locus of immunoglobulin in the typical translocation occurred in FL: t (14, 18, 72). In 60-90% of NHL cases, mentioned translocation and the placement of the Bcl-2 gene under the control of the enhancer region of IgH is observed (73, 74), whereas upregulation of Bcl-2 in the NHL without this translocation also with increasing relapse of the disease and mortality rate are associated (75).

#### Navitoclax

Navitoclax (ABT-263) is used as an inhibitor of the anti-apoptotic proteins of Bcl-xL, Bcl-2, Bcl-w, and Mcl-1/A1 in hematological malignancies, alone or combination with other apoptotic inhibitors. Navitoclax competitively averts Bcl-2 pro-apoptotic family members from being interrupted by Bcl-xL or Bcl-2 and thereby activating the intrinsic apoptotic pathway (76). In general, pre-clinical and clinical results have displayed strong Navitoclax activity in acute and chronic lymphocytic leukemia (77–79).

#### Venetoclax

Venetoclax (ABT-199, GDC-0199) is another selective Bcl-2 inhibitor that has safety and noteworthy activity in patients with different subtypes of NHL (80). In previous studies, Venetoclax showed notable activity in multiple subtypes of NHL, such as MCL, FL, and DLBCL.

### Checkpoint Inhibitors

Programmed death-1 (PD-1) is an inhibitory receptor expressed by active T cells that upon binding to its corresponding ligands, PD-L1/PD-L2 leads to suppression of T cell-induced immune responses and restriction of autoimmunity (81). Tumors often elude immune monitoring by up-regulating the PD-1 and/or PD-L1 level on tumor cells and tumor-associated immune cells (82). Recent studies have shown that PD-1 signaling, which is currently considered as one of the prominent mechanisms of immune escape, preferentially dephosphorylates and inhibits the co-stimulatory molecule CD28 (83). Many tumors, through overexpression of PDL-1, reduce the cytotoxic function of tumor-infiltrating T lymphocytes and thus escape immune surveillance. In some subset of patients with DLBCL, the PD-1 ligand gene amplification and PD-L1 overexpression have been observed in tumor cells and tumor-associated macrophages (84) so that after standard treatment, survival is attenuated significantly (85). In addition, overexpression of PD-1 has been observed in CD4^+^ tumor-infiltrating lymphocytes (TIL) in FL (86). Therefore, PD-1 inhibitors have been developed to disrupt this pathway and increase immune activity for the clinical advantage (87).

#### Durvalumab

Durvalumab is an anti-PD-L1 mAb that enhances anti-tumor immune responses by suppressing the interaction of PD-1 with PD-L1 (88). Data from previous studies in murine lymphoma models showed significant antitumor activity of Ibrutinib with the anti-PD-L1 Ab (89).

#### Nivolumab

Nivolumab is an anti-PD-1 Ab (a fully human IgG4 mAb) which activates T cell signaling through the PD-1 blockade, and thus enhances the anti-tumor response. Some studies propose that this drug may be beneficial for patients with relapsed FL after discontinuation of previous treatments (90).

#### Pembrolizumab

Pembrolizumab (formerly lambrolizumab) is a humanized mAb that targets the interaction between PD-1 and PD-L1/PD-L2 (91). The clinical effects of Pembrolizumab on Hodgkin’s lymphoma (HL) are significant, whereas the results are different in NHL. Subtypes of the NHL such as Primary mediastinal B cell lymphoma (PMBCL), that share genetic characteristics with HL, like chromosome 9p24.1 alterations and increased expression of PD-L1, have shown favorable responses in early-phase experiments (92). Pembrolizumab has been shown to potentiate the T lymphocytes’ immune responses in cultured blood cells from cancer patients and healthy human donors. Besides, it greatly modulates the levels of cytokines such as TNF-α, IFN-γ, and IL-2. Pembrolizumab does not induce cell-dependent cytotoxicity (CDC) or ADCC, and nonspecific T cell activation (93, 94).

#### Pidilizumab

Pidilizumab (CT-011) is a recombinant human IgG1 Kappa mAb binding to PD-1. Pidilizumab treatment is safe and tolerable, and its clinical activity has been recently demonstrated in DLBCL. PD-1 is an inhibitory receptor belonging to the B7 receptor family that is expressed on the myeloid cells and lymphocytes (95, 96) and by binding to the corresponding ligands (PD-L1 and PD-L2) adjust the immune response (97). In inflammatory conditions such as malignancy, continuous expression of PD-1 and its ligands by tumors leads to inhibition of the antitumor activity of tumor-infiltrating lymphocytes, T cell exhaustion, and immune escape (98). The binding of Pidilizumab to PD-1 attenuates the apoptotic process in this effector memory T cells. Pidilizumab upregulates the expression level of Bcl-xL protein by inducing the P13K signaling pathway, thus protecting effector/memory (CD45RO^+^) lymphocytes from apoptosis (99). Also, Pidilizumab may increase the antitumor activity of NK cells through the P13K signaling pathway.

## Combination Studies

The therapeutic effect of Rituximab in combination with Bendamustine was tested *in vitro* in primary CLL and CD20-positive DLBCL (100) and *in vivo* in a model of Burkitt’s lymphoma (BL) (101). Bendamustine is currently used to treat some hematological tumors, including the Rituximab-resistant and indolent NHL (102).

The Epratuzumab plus Rituximab can exert greater therapeutic impacts than any of the drugs alone in low-grade FL and DLBCL, which is characterized by a significant improvement in CR rate (103).

In a phase II study, MOR208 with Lenalidomide was evaluated in patients with R/R DLBCL (L-MIND study) (104).

Otlertuzumab in combination with Rituximab as well as chemotherapeutic drugs increased apoptosis in human B cell tumors. The use of TRU-016 and bendamustine also significantly delayed tumor growth *in vivo* and improved survival in xenograft lymphoma models compared with single agent therapy (105).

Inotuzumab ozogamicin (IO) has been tested in clinical trials along with Rituximab (106, 107), as well as in combination with Rituximab plus chemotherapy to treat NHL (108). The combination therapy with IO and Rituximab provides non-overlapping and distinct antitumor mechanisms including Ab-dependent cytotoxicity, cytotoxic agent delivery by IO, complement-dependent cytotoxicity, and induction of apitosis by Rituximab.

It has been shown that Ibrutinib together with ACY1215, a selective histone deacetylase-6 inhibitor, synergistically resulted in increased apoptosis in MCL cell lines compared to the monotherapy (109). Moreover, Ibrutinib in combination with Bortezomib raised cytotoxicity in DLBCL and MCL cells through mitochondrial damage and apoptosis (110). Also, the combination treatment of Ibrutinib and lenalidomide synergistically resulted in the eradication of ABC-type DLBCL cells (111). Ibrutinib along with Idelalisib synergistically disrupt BCR-stimulated integrin-mediated adhesion and inhibit the migration of CLL and MCL cells, supporting the justification for combination therapy (112).

The evaluation of Navitoclax in combination with Rituximab in patients with R/R CD20^+^ lymphoid malignancies and patients with previously untreated B-cell CLL exhibited synergistic antitumor activity and good tolerability (113, 114). In another study, the effects of combining Bendamustine or Rituximab with Navitoclax in the treatment of several NHL tumors were investigated. The results showed that Navitoclax enhanced the response of NHL tumors to Bendamustine in mouse xenografts and the addition of Rituximab increased the effectiveness of Bendamustine. In fact, treatment with Bendamustine increased p53 levels in Granta-519 tumors, thereby increasing the cleavage of caspase-3 and inducing apoptosis (115).

Previous studies have shown that Syk inhibitors (R406), Btk inhibitors (Ibrutinib), PI3K inhibitors (Idelalisib, Copanlisib, ACP-319, and KA2237), and other kinase inhibitors alone or in combination with Venetoclax significantly reduce the expression of BCL2 proteins *in vitro* and exerted synergistic killing impacts on lymphoma cells (116, 117). Clinical studies have confirmed that the combination of Ventoclax with Rituximab and Bendamustine can illustrate synergistic effects and significantly increase ORR and complete response (CR) rate in patients with DLBCL, FL, and MZL. Preclinical studies have also shown that Venetoclax along with Rituximab leads to complete tumor regression (100%) in R/R FL xenograft models (118). A phase II clinical trial investigated the combined influence of Venetoclax and Ibrutinib in patients with previously untreated or RR MCL. After completing the treatment, approximately 70% of the patients were negative for MRD (minimal residual disease) and indicated a CR of 67% (119).

## Manufacturing and Delivery of CAR‐T Cells

The production processes of different CAR-T cell lines are similar for the treatment of lymphoma. Peripheral blood mononuclear cells (PBMCs) are collected from blood, through the central or peripheral venous during outpatient leukapheresis. In the next step, PMBCs are transported to the production site at a temperature of 1-10°C and after being selected using density gradient T‐ lymphocytes or magnetic beads, they are activated by provoking their T cell receptor (TCR) (120). A viral transfer vector (retrovirus or lentivirus) then transfects the CAR gene to the activated T cell genome, causing the modified T cell to express the CAR molecule forever (121). Finally, after the T cells have spread in the flask, culture bags, or bioreactor systems, the CAR-T cell product is frozen and sent to the treatment site. The manufacturing process of a CAR-T cell product takes an average of 10-21 days, depending on the sort of CAR-T product. Before injection, lymphodepleting chemotherapy such as cyclophosphamide and fludarabine by depletion of regulatory T cells allow incoming T cells to proliferate and expand (**Figure 1**) (122).

**Figure 1:** Characteristic of CAR-T cells and their isolation, engineering, transfection, and expansion in patients with NHL. The first stage of CAR-T cell engineering is leukapheresis in which leukocytes are collected through central or peripheral venous (Stage 1). Then, PBMCs are purified among collected leukocytes (Stage 2). Next, density gradient or magnetic beads are used to purify T cells among collected PBMCs. Also, T cells get activated by provoking their TCRs (Stage 3). Viral transfection methods using viral vectors such as retrovirus or lentivirus are the next steps (Stage 4). The next step is done ex-vivo in which the cells are directed to be expanded (stage 5). In the last stage, modified CAR-T cells are expanded by culturing or bioreactor system and were injected into the same patients (step 6). Various antigens used as CAR-T cells’ targets in NHL have been shown. CAR, chimeric antigen receptor; PBMC, peripheral blood mononuclear cell; TCR, T-cell receptor.

## CAR Structure

A CAR molecule consists of three major domains: antigen recognition, transmembrane, and intracellular domain. The antigen detection domain consists of a single-chain variable fragment (scFv) containing the variable regions of the light and heavy chains of a monoclonal antibody against a certain antigen (eg CD19) (123). scFv, which partially modulates the function and safety of CAR-T cells, is attached to the membrane domain by a spaced region derived from IgG4 or CD8 molecules (124). Signal transduction due to antigen binding occurs *via* scFv to the intracellular domain (s). Ultimately, the intracellular domain, which usually includes the CD3ζ chain, acts as a signaling domain. The existence of additional costimulatory domains in CARs preserves T cell proliferation, activation, and survival (125). The CARs design has developed dramatically over the years.

The first-generation CAR-T is made of a CD3ζ chain as a crucial transmitter of endogenous TCR signals. After successful results in preclinical trials, the drug entered into phase 1 clinical trials for lymphoma, leukemia, neuroblastoma, ovarian cancer, etc (126). The variable regions of light and heavy chains of the B-cell receptor are called scFv, which, after fusion with ζ chain of the TCR or CD3 domain, form the activating receptor molecules that are non-HLA-restricted. By specifically targeting tumor cells, these molecules accelerate the detection of antigen by T cells and increase cytotoxicity (127). The artificial signaling receptors, CAR or chimeric receptors, and their synthesis method are called the T body approach (128).

The second-generation CAR-T cell therapy was established after the success of first-generation CARs in phase 1 clinical trials. Initially, these CAR-T cells were utilized in patients with recurrent B−cell ALL, and they created a more significant anti-leukemic response with a full recovery rate of up to 90%. The second-generation CARs contain a CD3ζ chain and an intracellular signaling domain of various co-stimulatory molecules, such as 4-1BB (CD137), CD28, OX40 (CD134), and induction T cell stimulator (ICOS or CD278) (129). For example, second-generation anti-CD19 CAR-T cells were constructed from a 4−1BB or CD28 costimulatory domain bound to the CD3 domain (130) which in patients with R/R B-cell malignancies produces remarkable complete response (CR) rates (131). While 4-1BB-based CARs accelerate the accumulation of T cells, CD28-specific CAR-T cells significantly increase effector T cells’ activity (132).

Third-generation CARs consist of two signaling domains and a CD3ζ chain such as the CD3ζ-CD28-OX40, which, compared to second-generation CARs, have increased activation signals, the length of the proliferation period, cytokine production, and effective anti-tumor activity in these cells (133). For example, a third-generation CAR consisting of α-CD19/CD3ζ/CD28/4−1BB segments dramatically increased the rate of complete recovery in patients with CLL by penetrating and lysing tumor cells (134).

Although all previous CARs have effectively contributed to T cell anti-cancer responses, they also have limitations, including degradation caused by antigen-negative cancer cells and the absence of antitumor action against solid tumors due to the broad phenotypic heterogeneity. These restrictions paved the way for the emergence and development of a new generation of CARs (135). Fourth-generation CARs, through the triggered expression of transgenic immunomodulators, such as IL−12, activates innate immune cells and thus increases T cell function, to lessen antigen-negative tumor cells in the designated lesion (134).

## Antigen Selection

The constant expression of B cell markers CD19, CD20, and CD22 in many B cell malignancies and previous reports of safety and efficacy of mAb against a mentioned surface antigen in these diseases have made them ideal targets for CAR-T cell therapy (25, 136). CAR therapy partially eliminates normal B cells because they also express most of the CAR-targeted lymphoma antigens, although this state can be compensated by intravenous immunoglobulin administration. Thus the use of more specific antigens that are limited to B cell malignancies as a target, compared with ordinary antigens, CD19/CD20/CD22, has fewer side effects. One of these alternative antigens is BCMA (B cell maturation antigen), which is expressed by the mature B cell subsets, plasma cells, and the light chain κ/λ of malignant B cells. In T cell lymphoma, the expression of many target antigens is common between malignant and normal T cells, so finding the ideal target antigen is more challenging. This joint expression of antigen can disrupt CAR-Ts function, prevent them from proliferating and surviving, and lead to the extinction of normal peripheral T cells (**Figure 1**) (137).

## CAR-T Cells for NHL

Most CAR-T clinical trials for the treatment of B-cell lymphoma target the CD19 marker. Because the expression of this antigen is seen in all stages of B cell differentiation and most B cell lymphomas (138). Different types of scFv can be applied to target the CD19 antigen. SJ25c or FMC63 are two of the most widely used scFvs in clinical trials (139). In the primary clinical trials for lymphoma therapy, a first-generation CAR-T (FMC63 19z CAR-T) without the costimulatory domain was used with the targeting CD19 (140). In this trial, patients with R/R FL after lymphodepletion with fludarabine and injection of IL-2 subcutaneously were treated using the first-generation anti-CD19 CAR-Ts. Despite proving the safety and feasibility of this new method, the first generation of anti-CD19 CAR-T cells did not show significant antitumor effects (140). However, the use of the second generation anti-CD19 CAR-T-cells with a costimulatory domain (4-1BB, CD28, and ICOS) in preclinical studies have shown considerable anti-tumor impacts *in-vitro*/*in-vivo* (141). Recently, the use of second-generation CAR-Ts targeting CD19 with stimulatory domains of CD28/4-1BB has reported considerable outcomes in the treatment of B-cell lymphomas, particularly PMBCL, DLBCL, splenic marginal zone lymphoma (SMZL), FL, and MCL (142).

One of the most common forms of aggressive NHL is DLBCL, which accounts for approximately 40% of cases (143). The standard initial treatment is combination of a chemotherapy regimen, usually R-CHOP (Rituximab, Cyclophosphamide, Adriamycin, and prednisone) and immunotherapy for 6-8 courses (144). Treatment is usually poor in people with high-risk characteristics such as early relapse in less than a year, preliminary refractory disease, and single/double-hit lymphoma (145). The preparatory examination of anti-CD19 CAR-T cells provided promising therapeutic effects (146). Jensen et al. used CD20-targeted CAR-T cells to treat two patients with recurrent DLBCL who had previously undergone autologous hematopoietic stem cell transplantation. They did not observe any obvious toxicity or clinical complication in these patients after treatment (140). In another experiment, anti-CD19 CAR-T cells were used on several patients with advanced B cell malignancies. After treatment, complete remission (CR) was observed in 4 patients out of the total number of chemotherapy-refractory DLBCL patients (147). Besides, Stirrups et al. injected anti-CD19 CAR-T cells into several patients with large B cell lymphoma, including PMBCL and DLBCL. After treatment, the analysis of patients showed that 28% of them had PR and 54% had CR (148).

Follicular lymphoma is the most common indolent lymphoma that accounts for 10-20% of NHL. The genetic characteristic of FL is the translocation of t (14; 18) (q32; q21), which leads to overexpression of BCL-2 protein and disruption of the apoptotic program of the germination center (149). Besides, FLs show additional genetic changes such as mutations, losses, or gains in genes such as EPHA7, MLL2, CREBBP, CREBBP, TNFRSF14, EZH2, BCL6, and so on (150). Many patients with FL remain asymptomatic despite the widespread disease. About 10-15% of FLs are diagnosed in the primary stages and the rest in advanced stages III and IV (150). Advanced-stage III/IV follicular lymphoma becomes resistant to chemotherapy and may convert into a more aggressive subtype of the NHL, such as DLBCL (151). The biological nature of this malignancy is such that eventually, most patients experience relapsing stages of the disease or resistance to treatment. Therefore, CAR-T cell therapy can be considered an attractive treatment approach. Schuster et al. used CTL019 in a phase IIa study in patients with FL and showed that disease progression in these patients occurred 2 years after remedy with two or more treatment lines (152). Furthermore, In another study, a patient with R/R acute B cell lymphoblastic lymphoma and Li-Fraumeni syndrome (LFS) received dual specific CD19/CD22-targeted CAR-T cells. After that, several parameters showed complete relief of the tumor and negative MRD (153). Also, a group of researchers used KTEC19 consisting of FMC-63 (a single-chain Ab in the extracellular region) that detect CD19 at the tumor cell surface to treat aggressive and refractory B-NHL patients (154).

Mantle cell lymphoma is an uncommon form of NHL with unique immunophenotypic and clinical features that accounts for about 6% of NHL cases. In MCL cells, due to chromosomal translocation t (11:14), the expression of cyclin D1 is greatly increased (155). The standard therapy is induction chemotherapy with or without autologous grafting to integrate into responsive patients followed by maintenance therapy with anti-CD20 mAb therapy. This method can lead to lasting improvement but does not seem to be the mainstay of treatment, and the prognosis for patients with early recurrence can be poor (156). One way to diagnose this malignancy, like other forms of NHL, is to examine the CD19 expression. CAR-T cell therapy is an effective way to treat MCL and to some extent makes the disease a treatable condition. In a clinical trial, the effect of third-generation CD20-directed CAR-T cells on several patients with MCL and relapsed indolent B cells was evaluated. The results showed that this treatment was well tolerated, although disease relapsed in one of the patients one year after injection (129).

Burkitt’s lymphoma is one of the most common forms of NHL in children, and about 10% of patients with a poor prognosis, relapse even after vigorous chemotherapy. In a recent study, an eight-year-old child was initially treated with CD19-specific CAR-T cell but showed progressive disease (PD) and illustrated no clear response to cell therapy. CD22-specific CAR-T cells were then injected into the child, but recurrence of the disease was observed. Finally, CD20 CAR-T cell treatment resulted in the achievement of CR (157). Besides, CAR-T cell therapy targeting tyrosine kinase-like orphan receptor (ROR1) and CD23 has yielded promising results in advancing R/R NHL therapy (**Figure 2**) (158).

**Figure 2:** Generations of CAR-T cells along with allogenic, transgenic, bispecific, and armored CAR-T cells. In the upper quadrant, allogeneic and transgenic CAR-T cells are seen. Allogeneic CAR-T cells are seen in patients that have allogeneic HSCT and can be either donor- or recipient-derived. On the other hand, transgenic CAR-T cells are engineered CAR-T cells that have been made by transfection of a special gene to encode the surface receptor of CAR-T cells. In the middle quadrant, three generations of CAR-T cells are shown. Besides, bispecific CAR-T cells are engineered to target two different targets simultaneously. In the lower quadrant, armored CAR-T cells which have been potentiated by secreting cytokines and chemokines are seen. HSCT, hematopoietic stem-cell transplantation; CCR2, chemokine receptor 2.

## Current CAR T-Cell Products

### Anti-CD19 CAR-T Cell Therapy for B-Cell NHL

Numerous studies have been actively conducted since 2010 when the first case of anti-CD19 CAR-T cell treatment was reported, until 2017 when the first approval for this product was received by the US FDA (142, 152, 159). To date, several CD19-specific CAR-T cell therapies have been tested in B cell malignancies. Among these CAR-T products, tisagenlecleucel (tisa-cel), axicabtagene-ciloleucel (axi-cel), and lisocabtagene-maraleucel (liso-cel) in a relatively wide range on patients with aggressive B cell lymphomas especially DLBCL are being tested (160). To produce Axi-cel, a retroviral vector, and the co-stimulatory/transmembrane domains of CD28 are used (161). Tisa-cel is generated using a lentiviral vector, a CD8-α transmembrane domain, and a 4-1BB co-stimulatory domain (162). Liso-cel is made with a lentiviral vector, a CD28 transmembrane domain, and a co-stimulatory domain of 4-1BB. The manufacturing and time required to produce distinct products are different. For example, liso-cel is made up of equal proportions of CD4^+^ and CD8^+^ CAR-T cells, while both tisa-cel and axi-cel are produced from bulk T cells in which the cell dose varies from patient to patient. The turnaround time (from leukapheresis to product accessibility) of both tisa-cel and Liso-cel is approximately 24 days, while in Axi-cel it is approximately 17 days (162, 163).

### Axicabtagene-Ciloleucel (KTE‐CD19, Axi-cel)

Axi-cel is a second-generation CAR-T with a CD28 domain embedded in its structure and was first developed by the National Cancer Institute (NCI) researchers. Kite Pharma, Daiichi Sankyo, and Gilead Sciences conducted a fundamental phase I/II study of axi-cel in patients with PMBCL, transformed FL, and high grade and R/R DLBCL called the ZUMA-1 test (NCT02348216) (164, 165).

### Tisagenlecleucel (CTL019)

Tisa-cel was the second CAR-T cell product for invasive B cell lymphoma that received FDA approval based on the JULIET trial. In an international phase 2 JULIET study, patients with DLBCL, HGBCL (double-hit lymphoma), and transformed FL had received two or more treatment lines and were chemotherapy or multiply refractory/relapsed or unqualified for autologous stem cell transplantation (166). This product is the first CAR-T cell to be approved by the FDA in 2017 for the treatment of pediatric B-cell acute lymphoblastic leukemia (B-ALL) (167). It should be noted that this research was first conducted by researchers at the University of Pennsylvania (UPenn) in assistance with Novartis.

### Lisocabtagene Maraleucel (JCAR017, Liso-cel)

Liso-cel is the third major CD19-specific CAR-T cell product and is awaiting FDA approval based on TRANSCEND-NHL-001 data, a monolithic pivotal project that studied patients with DLBCL NOS, HGBCL (double-hit lymphoma), transformed indolent B-cell lymphomas, follicular lymphoma grade 3B, and PMBCL (163). The researchers at the Memorial Sloan Kettering Cancer Center, Fred Hutchinson Cancer Research Center (FHCRC), and Seattle Children’s Research Institute founded a venture, Juno Therapeutics, performed several clinical trials on anti-CD19 CAR-T cell products including JCAR014/015/017/021, and so on. In the next phase clinical trial, JCAR017 (lisocabtagene-maraleucel, liso-cel) was evaluated in patients with B-NHL. Liso-cel is a second-generation anti-CD19 CAR-T cell with a costimulatory domain of 4-1BB and is made from an isolated subset of CD4^+^ and CD8^+^ cells with a 1:1 CD4/8 ratio. The results of researchers’ preclinical studies at the FHCRC reported that CAR-T produced from different T cell subsets showed distinct activity *in-vivo* (168). For example, the direct anti-tumor activity of CD8^+^ central memory (CD8^+^ CM)-CAR-T is much stronger than that of CD4^+^ CAR-T. CD4 ^+^ CAR-T cells lead to a synergistic increase of proliferation after CD8^+^ CM-CAR-T injection by producing several inflammatory cytokines (**Table 2**) (160).

**Table 2:** The clinical trials of CD19-targeted CAR T cells.

No. of patients/age (years)	Disease/No. of patients	CAR generation	Co-stimulatory domain	Injected CAR T cell dose	Result	Ref
4 (n/a)	FL:2	I	None	1−2×10^9^/m^2^	2 PD	(140)
1 (n/a)	FL	II	CD28	1−3×10^8^	1 PR	(142)
6 (46–59)	NHL	I+II	None/	2−20×10^7^/m^2^	2 SD, 4 NR	(169)
			CD28			
3 (64–77)	CLL	II	4-1BB	1.4×10^5^/kg −1.6×10^7^/kg	2 CR, 1 PR	(170, 171)
8 (47–63)	CLL: 4,	II	CD28	0.3–2.8×10^7^/kg	CLL: 1 CR, 2 PR, 1 SD	(172)
	FL: 3 SMZL:1				FL: 2 PR, 1 NE	
					SMZ: 1 PR	
10 (44–66)	CLL: 4 DLBCL: 2	II	CD28	0.4–7.8×10^6^/kg	CLL: 1 CR, 1 SD, 2 PD; DLBCL:	(173)
	MCL: 4				2 SD;	
					MCL: 3 SD, 1 PR	
8 (9–59)	ALL: 4	II	CD28	1.5−12×10^7^/m^2^	3 CR, 1 PD	(174)
	CLL: 4				1 PR, 1 SD, 2 PD	
14 (51–78)	CLL	II	4-1BB	0.14−11×10^8^	4 CR, 4 PR, 6 NR	(175)
21 (1–30)	ALL: 20	II	CD28	1−3×10^6^/kg	ALL: 14 CR, 3 SD, 3 PD	(176)
	DLBCL: 1				DLBCL: 1 PD	
15 (30–68)	CLL: 4 DLBCL: 5	II	CD28	1–5×10^6^/kg	CLL: 3 CR, 1 PR; DLBCL: 2 CR, 2	(147)
	SMZL: 1 PMBCL: 4				PR, 1 NE; SMZL: 1 PR; PMBCL;	
	LG-NHL: 1				2 CR, 1 SD, 1 NE; LG-NHL: 1 CR	
20 (25–68)	CLL: 5 DLBCL: 5	II	CD28	0.4–8.2×106/kg	CLL: 1 CR, 1 PR, 1 SD, 2	(177)
	MCL: 5				PD; DLBCL: 1 CR, 3 SD, 1	
	ALL: 5				PD; MCL: 1 PR, 4 SD	
					ALL: 4 CR, 1 PD	
32 (36–70)	NHL	II	4-1BB	0.2−20×10^6^/kg	11 CR, 9 PR, 10 NR, 2 NE	(178)
16 (23–75)	DLBCL: 11 MCL: 5	I+II	None/	2.5−20×10^7^	DLBCL: 8 CR, 2 PR, 1 PD; MCL:	(179)
			CD28		5 CR	
26 (23–61)	ALL: 17	II	CD28	Varying doses	9 CR, 2 SD, 6 PD	(180)
	FL: 3 DLBCL: 4				FL: 3, DLBCL: 4,	
	MCL: 1				MCL: 1, HL: 1	
	HL: 1				DLBCL: 2 CR, 1 SD, 1 PD; FL: 3	
					CR; MCL: 1 CR;	
					HL: 1 CR	
7 (29–69)	DLBCL	II	CD28	2×10^6^/kg	4CR, 1 PR, 1 SD, 1n/A	(165)
24 (40–73)	CLL	II	4-1BB	0.2−20×10^6^/kg	CR+PR: 17, 7 NR	(181)
101 (23–76)	DLBCL: 77		CD28	2×10^6^/kg	38 CR, 25 PR, SD 9, PD 4; NE: 1	(178)
	PBMCL or FL: 24				17 CR, 3 PR, 2 SD, 1 PD, 1 NE	
14 (25–77)	DLBCL	II	4-1BB	1−5×10^6^	6 CR, 1 PR, 7 NR	(152)
14 (43–72)	FL				10 CR, 1 PR, 3 NR	
15 (24–71)	ALL: 4 CLL: 2	III	CD28+4–1BB	2−20×10^7^/m2	ALL: 2 CR, 2 PD;	(182)
	DLBCL: 6 MCL: 2				CLL: 1 CR, 1 SD; DLBCL: 3 CR, 3	
	FL-Burkitt: 1				PD; MCL: 1 SD, 1 PD; FL-Burkitt:	
					1 PD	
16 (16–75)	DLBCL: 11 ALL:2	II+III	CD28/	2−40×10^6^/m2, 0.05–	DLBCL: 6 CR, 2 PR, 2 SD, 1	(183)
	BCLU: 1 LBL: 1		CD28+4–1BB	1.25×10^6^/kg	NR; ALL: 1 PR, 1 NR; CLL:	
	CLL: 1				1 NR; BCLU: 1 CR;	
					LBL: 1 CR	

ALL, acute lymphoblastic leukaemia; lymphoma unclassified; CLL, chronic lymphocytic leukaemia; CR, complete remission; DLBCL, diffuse large B-cell lymphoma; EP, electroporation; FL, follicular lymphoma; Gen, CAR generation; HL, Hodgkin’s lymphoma; LBL, lymphoblastic lymphoma; LG, low grade; MCL, mantle cell lymphoma; n/a, not assessed; NE, not evaluable; NHL, non-Hodgkin’s lymphoma; NR, no response; PD, progressive disease; PMBCL, primary mediastinal B cell lymphoma; PR, partial response; SD, stable disease; SB, Sleeping Beauty; SMLZ, splenic marginal zone lymphoma.

### Novel CAR-T Cells in NHL

Although the excitement of using CD19 CAR-T cells was initially significant in patients with R/R NHL, the (progression-free survival) PFS rate ranges between 30- 50%, and for those who do not receive CAR-T treatment, the results were unpleasant. According to studies, mechanisms such as lack of CAR-T durability, loss of CD19 antigen, and the presence of immune checkpoint molecules in tumor cells can cause recurrence of malignancies (184, 185). Several new clinical structures are currently being developed to remove these restrictions.

### Bispecific CARs or Dual Targeted CAR-T Cells

A bispecific receptor consists of two distinguished antigen recognition domains that bind to two separate intracellular domains and are expressed as tandem scFvs in one CAR, or as two different CARs on T cell surface. At current, CD19/CD20-bispecific CAR-T cells have been presented as a new synthetic molecule that, after recognition and binding to target tumor antigens on the surface of malignant cells, can establish a synergistic cascade of executive molecules (186). If one of the target molecules is not available to CAR T cells for reasons such as removal or mutation of the target antigen on malignant cells, a dual-function machine can largely prevent tumor escape. Thus, the bispecific CAR retains the cytolytic property of T cells (184). In addition to the mentioned CARs molecule, several other bispecific CARs including CD20/CD19 and CD20/CD3 have also been preclinically studied (187, 188).

### Inhibitory CARs (I−CARs)

The interaction of PD-1 receptors with PD-L1 inhibits the activity of T cells and is one of the mechanisms of escape from the immune system that promotes the survival of malignant diseases. This pathway is thought to play a key role in tumor escape from CAR-T cells, so treatments combining PD-1 inhibition with CAR-T cell therapy are being studied. In a recent study, Pembrolizumab was used as an immune checkpoint inhibitor (anti-PD1) at various intervals after CART19 treatment, including during early progressed or late relapsed of NHL to inhibit T cell exhaustion (189). Besides, Jacobson et al. showed that blockade of PD-L1 with the anti-PD-L1 antibody atezolizumab (atezo) significantly increased the efficacy and safety of ZUMA-6 in refractory DLBCL patients (190). It has already been shown that CTLA-4-/PD-1- based I-CARs can significantly control cytokine secretion, cytotoxicity, and proliferation induced by activating chimeric receptor or endogenous TCR (191). I-CARs control CAR T cell function by inhibitory receptors. I-CARs differentiate between normal and cancer cells by inhibiting the activator CAR response to antigens expressed only by normal cells (192). Therefore, the design of I-CAR using PD-1 and CTLA-4 surface antigen detection domains to regulate T cell response and prevent T cell inhibition physiology in mouse models has been confirmed. However, the use of this technique in mice lacking CTLA-4 and PD-1 receptors leads to severe systemic autoimmune diseases such as glomerulonephritis and arthritis (193, 194).

### Armored CAR-T Cells

Inducing the expression of an extra transgene - along with CAR – by effective T cells is one of the recent strategies to enhance CAR-T cells effector functions and control the immunosuppression caused by the tumor microenvironment. TRUCKs (T cells redirected for universal cytokine killing) are examples of armored CAR-T cells that transgenic cytokines (IL-12/-15/-18) produced by them accumulate in malignant tissue and show beneficial effects (195–197). Besides, some modifications allow armored CAR-T cells to express a ligand for costimulation molecules. Batlevi and colleagues used different doses of 19-28z/4-1BB-L CAR-T cells in phase I clinical trial to treat patients with CLL or NHL (198). Furthermore, in other studies, CAR-T cells were modified to deal with immunosuppressive signals. For example, CD19-targeted CAR-T cells with co-expressing of the chimeric switch receptor of PD-1/CD28 were examined for the treatment of patients with R/R DLBCL in phase I clinical trial (199). Also, the direct embedding of anti-PD-1 or anti-PD-L1 blockers in CAR-T cells can clearly illustrate the combined anti-tumor effects of CAR-T cells with checkpoint inhibitory antibodies (200).

### Allogeneic CAR-T Cells

To prevent the use of patient-derived inefficient T cells and reduce the cost/time of producing products, healthy donors-derived allogeneic CAR-T cells can be used. Because allogeneic products can cause graft versus host disease (GVHD) as well as CAR T cell rejection, strategies should be used to minimize donor-derived T cells alloreactivity before using off-shelf products. Recently, gene-editing technologies have been utilized to forbid the endogenous TCR expression on modified T cells. Several methods can be used to disrupt the TCR alpha constant (TRAC) gene, such as the CRISPR/Cas9 system, transcription activator-like effector nucleases (TALEN), and zinc finger nucleases (ZFN) (201). The universal CD19-targeted CAR-T cell product (UCART19) was produced following the simultaneous introduction of CAR and TCR knockout to prevent GVHD and CD52 suppression to induce resistance to anti-CD52 Ab to reduce the likelihood of UCART19 rejection in allogeneic T cells (202). ALLO-501 is an anti-CD19 allogeneic CAR-T (AlloCAR T™) with the same structure as UCART19, which has recently undergone clinical trials in the ALPHA study for the treatment of FL and R/R DLBCL. PBCAR0191 is another allogeneic CD19-directed CAR-T cells produced by using a single-stage TCR knock-out and CAR knock-in, and its antitumor effects have been demonstrated in a phase 1 trial in patients with NHL (203).

## Other Targets Against NHL

Sometimes mutations in the CD19 antigen or the downregulation/disappearance of this antigen from the surface of malignant lymphocytes lead to tumor escape and resistance/refractory to CD19-targeted CAR-T treatment in patients (204). According to recent studies, 40% of reported recurrences are due to epitope loss (205, 206). Therefore, alternative markers such as CD20, CD22, etc. with higher expression in B-NHL and B-ALL, respectively, can be used as a target for T cell therapies (207, 208). In the FHCRC phase-I experiment, third-generation anti-CD20 CAR-T cells containing CD28 and 4-1BB domains were used to treat MCLs and intolerant B-cell lymphomas. In this section, new studies of CAR-T cell therapy, which recognize different CAR-T cells and intensifies tumor cell death, are reviewed.

### CD20 CAR-T Cell Therapy

CD20 is a non-glycosylated membrane phosphoprotein that is highly expressed not only in normal B cells but also on the surface of malignant B cells (209). CD20 is expressed by CLL, all NHL cases, and about 40% of precursor B-ALL (210). Recently, Xu et al. evaluated the cytotoxicity effect of CD20-specific CAR-T cells on B cell malignancy using *in vitro/in vivo* true lytic ability, CD107a degranulation, and production of proinflammatory cytokines. They also used histone deacetylase inhibitors (HDACi) to increase CD20 marker expression on the surface of B- malignant cells by inducing H3K9 acetylation at the CD20 promoter region. The final results showed that the cytotoxicity of CD20-specific CAR-T cells in malignant B cells treated with HDACi was significantly increased compared to the untreated state (211).

### CD30 CAR-T Cell Therapy

CD30 (TNFRSF8), a cell membrane protein and tumor marker belonging to the TNF receptor family, is found on the surface of NHL cells including DLBCL, anaplastic large cell lymphoma (ALCL), PMBCL (212), adult T-cell leukemia/lymphoma (213), and peripheral T cell lymphoma (PTCL) (214), as well as in HL, and rare solid tumors (215). So far, this antigen has been widely used as a potential target for antibody-based therapy. One of the most notable results was obtained after treatment of ALCL and HL with an ADC-targeted CD30 (Brentuximab-vedotin/BV) (216). Afterward, CAR-T cells were explored to overcome the challenges posed by antibody-based therapy, such as low tumor penetration and inadequate response durability (217). Recently, the effect of immunotherapy with second CD30-targeted CAR-T cells has been demonstrated in preclinical models and clinical trials. However, after this treatment, no optimal response was observed in the patients, as most of them showed stable disease after multiple CAR-T cell injections. Besides, extra-nodal lesions showed a weaker response than lymph nodes, and T cells lasted only about two months after infusion (218–221). Thus, Guercio et al. demonstrated that using a new third-generation structure designed with the novel scFv, a combination of OX40 and CD28 costimulatory molecules, as well as the addition of the production process of IL-7 and -15, resulted in prolonged persistence and high proliferation of T cells, and immunological memory to prevent lymphoma recurrence (222).

### CD37 CAR-T Cell Therapy

CD37 is a tetraspanin protein that is widely expressed in all types of B-NHL (223). Its biological function is not completely understood, but it may be associated with apoptotic signals and survival as well as tumor suppression (224). Accordingly, CD37 is a potential target for B cell malignancies immunotherapy. So far, several anti-CD37 therapeutic agents have been investigated in phase 1 and 2 trials including a targeting peptide (Otlertuzumab), a mAb (BI836826), a radioimmunoconjugate (Betalutin; ^177^ Lu-lilotomab-satetraxetan), and antibodies-drug conjugate (AGS67E and IMGN529) (225, 226). The preclinical development and efficacy of anti-CD37 CAR-T cells have been recently demonstrated in T- and B cell malignancies (227). The effect and specificity of CD37 CAR-T cells against B-cell lymphoma have already been demonstrated in the mouse lymphoma xenograft models and *in vitro*. It has also been observed that CD37-expressing tumor cells, do not resist CD37 CAR-T cells (228). Koksal et al. developed a second-generation CD37-targeted CAR structure and compared its performance on T cell function in different B lymphoma cell lines with anti-CD19 CAR-T cells. They showed that in one xenograft model of aggressive B-cell lymphoma, both CAR-T cells were equally capable of controlling tumor growth, but in the second xenograft model, using the U2932, a CD19- subpopulation of lymphoma cells, CD37 CAR-T cells dramatically controlled the survival and tumor growth, while CD19 CAR-T cells were much less effective. Overall, the results of their studies showed that CD37 CAR-T cells could be used to eradicate those B-cell lymphoma tumors in which CD19 antigen expression has been lost, and after further investigation for patients with R/R B- NHL (229).

### CD38 CAR-T Cell Therapy

CD38, like CD19 due to its wide distribution on B-NHL cells, is an ideal molecular target for the treatment of this malignancy and, as previously reported, so far, no side effects following treatment with anti-CD38 Ab in B cell lymphoma patients has been reported (230). Furthermore, several types of Ab or Anti-CD38 Ab have been used in the treatment of CD38^+^ malignancies (209, 231–233). Recently, Mihara et al. demonstrated that anti-CD38-CAR-T cells have potent cytotoxicity and eradicate B-NHL *in vitro* and *in vivo* (**Table 3**) (234).

**Table 3:** The clinical trials of CAR-T cell therapies in T-NHL.

NCT	Study phase	Type	Disease
NCT03081910	1	CD5 CAR-T	R/R lymphoma or leukemia
NCT02963038	I+II	CD19 CAR T	B-NHL+ B-ALL
NCT03068416	II	CD19 CAR T	B-NHL + B-ALL
NCT03146533	I+II	CD19 CAR T	B-NHL
NCT02132624	I	CD19 CAR T	B-NHL
NCT03105336	II	CD19 CAR T	R/R Indolent B‐NHL
NCT03676504	I+II	CD19 CAR T	B-NHL + B-ALL
NCT01853631	I	CD19 CAR T	B-NHL + B-ALL
NCT03277729	I+II	CD20 CAR T	R/R B‐NHL
NCT03019055	I	CD19/20 CAR T	R/R B‐NHL
NCT03448393	I	CD19/22 CAR T	R/R B‐NHL or ALL
NCT03233854	I	CD19/22 CAR T	R/R B‐NHL or ALL
NCT03330691	I+II	CD19/22 CAR T	R/R lymphoma
NCT02153580	I	CD19/EGFR CAR T	R/R B‐NHL
NCT03244306	I	CD22/EGFR CAR T	R/R lymphoma or leukemia
NCT02601313 (ZUMA-2)	II	Axi-cel	MCL
NCT03105336 (ZUMA-5)	II	Axi-cel	MZL, FL
NCT03624036 (ZUMA-8)	I+II	Axi-cel	CLL
NCT04162756 (ZUMA-18)	EA	Axi-cel	MCL
NCT02631044 (TRANSCEND-NHL-001)	I	Liso -cel	FL G3b, MCL
NCT03483103 (PILOT)	II	Liso -cel	FL G3b
NCT03744676 (OUTREACH)	II	Liso -cel	FL G3b
NCT03568461 (ELARA)	II	Tisa-cel	FL
NCT03331198 (TRANSCEND-CLL-004)	I+II	Liso-cel +/- ibrutinib	CLL
NCT03575351 (TRANSFORM)	III	Liso-cel *vs* ASCT	FL G3b
NCT03310619 (PLATFORM)	I+II	Liso-cel + CC-122	FL G3b
		Liso-cel + durvalumab	
NCT03049449	I	CD30 CAR T	R/R lymphoma
NCT02663297	I	CD30 CAR T	Lymphoma s/p auto SCT
NCT02917083	I	CD30 CAR T	R/R lymphoma
NCT02690545	I+II	CD30 CAR T	R/R lymphoma
NCT03602157	I	CD30/CCR4 CAR T	R/R lymphoma
NCT02917083	I	CD30 CAR T	R/R CD30^+^ HL and NHL
NCT03049449	I	CD30 CAR T	R/R CD30+ HL and NHL
NCT03383965	I	CD30 CAR T	R/R CD30+ HL and NHL
NCT02663297	I	CD30 CAR T	R/R CD30+ HL and NHL
NCT02690545	I+II	CD30 CAR T	R/R CD30+ HL and NHL
NCT02259556	I+II	CD30 CAR T	R/R CD30+ HL and NHL
NCT02958410	I+II	CD30 CAR T	R/R CD30+ HL and NHL

ALL, acute lymphoblastic leukemia; NHL, non-Hodgkin lymphoma; CAR, chimeric antigen receptor; HL, Hodgkin lymphoma; R/R, relapsed/refractory; EA, expanded access; G3b, grade 3b.

## CAR-T Cells Toxicities & Management

The observation of some life-menacing toxicities following the activation of the immune system with CAR-T cell therapy limits the widespread use of this therapeutic approach (235). It seems that the degree of toxicity created depends on various factors such as the type of vector, scFv, co-stimulatory domain, CAR-T cells’ dose, disease burden, and preconditioning regimen (7). Studies show that in practice, the incidence and severity of toxicity in CAR-T cell products with a CD28 costimulation domain are higher than products containing a 4-1BB domain. Because the CD28 domain leads to the fast and high expansion of CAR-T cells, while the 4-1BB domain leads to gradual expansion and long continuance (236). Cytokine release syndrome (CRS) and neurotoxicity are among the most common toxicities caused by CAR-T cell therapy (237). CRS is a systemic inflammatory response that happens after the secretion of inflammatory cytokines such as IL -1, 2, 6, 10, TNF-α, and IFN-γ from the immune cells and CAR-T cells (238). This toxicity can occur from a few hours to several days after the CAR-T cell inoculation. CRS is characterized by symptoms such as hypotension, high fever, hypoxia, sinus tachycardia, and organ dysfunction (239) and altered laboratory values include significant increases in ferritin, increased CRP, and low fibrinogen (240). Early detection and management are important because some reports indicate death from severe CRS (239). CRS is graded based on the degree of hypoxemia, hemodynamic instability, and organ injury (241, 242). Treatment of CRS depends on the intensity of the signs as well as the patient underlying diseases. Specialists recommend supportive and precise surveillance with fluids for grade 1 CRS. However, for higher-grade CRS, immunosuppressive agents are commonly employed (243). Because IL-6 plays a crucial role in the development of CRS, one of the IL-6 receptor blockers, tocilizumab, is used in patients with higher CRS (244). Corticosteroids are also applied in cases where tocilizumab is incapable to control the symptoms of severe CRS (242). Furthermore, CAR-T cells cause neurologic toxicity, which is called CAR-T cell-related encephalopathy syndrome or CRES and recently this term was replaced by “Immune effector cell-associated neurotoxicity syndrome (ICANS)” (245, 246). Neurotoxicity probably indicates the capability of CAR-T cells to infiltrate into the blood-brain barrier (242). This toxicity can lead to ataxia, mild cognitive defects, tremor, somnolence, dysphagia, obtundation, snoring, and seizures, as well as death in severe cases. The occurrence of neurotoxicity may be simultaneous or independent of CRS (247). Dexamethasone appears to penetrate the blood-brain barrier to some extent reversing neurological symptoms. However, it is unlikely that the monoclonal antibody tocilizumab will penetrate the blood-brain barrier (248). There have been no reports of tocilizumab being effective in this type of toxicity. According to previous studies, steroids are the mainstay of CRS treatment. Other complications of CAR-T cell therapy include infection and cytopenias. In addition, B cell aplasia leads to hypogammaglobulinemia and subsequent recurrent infections due to targeting CD19 present on B lymphocytes. Intravenous immunoglobulin administration in these patients largely helps to control the mentioned symptoms. Due to chemotherapy and malignancy, patients’ immune systems are significantly suppressed and they are prone to fungal, bacterial, and viral infections. Prophylactic antibiotics, antiviral and antifungal drugs are used to prevent the spread of infection in these patients (248). Anaphylaxis, tumor lysis syndrome, and hemophagocytic lymphohistiocytosis are among the less common complications after treatment with CAR-T cells (238).

## Future Directions

At present, anti-CD19 CAR-T cells created a sustainable recovery in 40% of chemotherapy-resistant DLBCL, HGBCL, and PMBCL patients who have not previously received any treatment options. Also, these products are currently used in patients with aggressive lymphoma who have relapsed after at least 2 previous treatment lines. Besides, clinical trials of anti-CD19 CAR-T cells in patients with DLBCL are being considered as a treatment option in the first recurrence. Currently, high-dose chemotherapy with ASCT has been considered as the second line of treatment for DLBCL, and about 20% of patients are treated with this method (249, 250). However, in many patients, due to resistance to chemotherapy, old age, and the presence of comorbidities diseases, there will be no necessary conditions for such treatment. Additional strategies are needed to overcome mechanisms of resistance to CD19 CAR-T cells, including T cell depletion, loss of target antigen, loss of continuance, and immune escape. Approaches such as combining CAR T cell products with immunomodulating drugs (251), tyrosine kinase inhibitors (252, 253), and immune checkpoint inhibitors (254) have shown promising results *in vitro*. Besides, the novel CAR structures, known as third-generation CARs, greatly enhance the activity of T cells (183). These CAR-T cells include 1) CAR-T cells that target several cancer antigens simultaneously, such as CD19 and CD22, which prevents antigen loss (255), 2) CAR-T cells that directly suppress immune checkpoints (254), 3) CAR-T cells that use gene editing to insert the CAR gene in a position that enhances activation and reduces T cell exhaustion (256), 4) CAR-T-cells secreting cytokines such as IL-12 which may impair the suppressive function of the tumor microenvironment (257, 258). Finally, new allogeneic products are likely to replace autologous CAR- T cells. Autologous T cell products have limitations such as poor T cell health derived from patients who have already received lymphoma treatments, the time-consuming production process in patients with R/R high-grade lymphoma, and costly process apheresis, bridging, and construction. Allogeneic CAR-T cells may overcome these barriers by using gene-editing technology by removing the T cell receptor from the healthy donor T cell by inserting the CAR gene against the target tumor antigen (259). Allogeneic CAR-T cells are presently being studied in early-stage clinical trials in lymphoma patients. Finally, the possibility of using CAR-T cell technology in T cell lymphoma and solid tumors is expanding. It is important to select a target antigen that is tumor-specific enough because less specific markers increase the destructive immunological attack on healthy tissues from which the malignancy has developed.

## Conclusion

The current advances in CAR-T cell therapy have presented us with highly efficient solutions aimed at treating patients with NHL. Although the efficacy of CAR-T cells has been proven in previous studies, it is still possible to further improve the effectiveness and speed up the response time. Besides, neurotoxicity and CRS induced by CAR-T treatment can cause considerable morbidity in patients receiving this type of treatment. Therefore, the use of new treatment strategies such as T cell engagers, targeted molecular therapies, checkpoint inhibitors, and antibody-drug compounds in the conjunction with CAR-T cell treatment not only reduces side effects but also generates positive changes in the treatment of hematologic malignancies like the NHL creates.

## Author Contributions

All authors contributed to the conception and the main idea of the work. FM, SI, HS, MA, KS, WS, WA, MM, NS, and AH drafted the main text, figures, and tables. M.J supervised the work and provided the comments and additional scientific information. MA, MY, RM, YP, and A.C-A also reviewed and revised the text. All authors contributed to the article and approved the submitted version.

## Funding

We would like to appreciation German Cancer Research Center (DKFZ) for their financial support.

## Conflict of Interest

The authors declare that the research was conducted in the absence of any commercial or financial relationships that could be construed as a potential conflict of interest.

## Abbreviations

CAR, chimeric antigen receptor; GvHD, graft-versus-host disease; NK cells, Natural killer cells; NHL, non-Hodgkin lymphomas; DLBCL, diffuse large B-cell lymphoma; FL, follicular lymphoma; ALL, lymphoblastic leukemia; CRS, cytokine release syndrome; RCC, renal cell carcinoma.

## References

[1] TsengC-HWangW-CChenC-YHsuH-JChenY-K. Clinical Manifestations of Oral Lymphomas–Retrospective Study of 15 Cases in a Taiwanese Population and a Review of 592 Cases From the Literature. J Formosan Med Assoc (2020) 120:361–70. 10.1016/j.jfma.2020.05.025 32505589

[2] VitoloUTrněnýMBeladaDBurkeJMCarellaAMChuaN. Obinutuzumab or Rituximab Plus Cyclophosphamide, Doxorubicin, Vincristine, and Prednisone in Previously Untreated Diffuse Large B-Cell Lymphoma. J Clin Oncol (2017) 35(31):3529–37. 10.1200/JCO.2017.73.3402 28796588

[3] CrumpMNeelapuSSFarooqUVan Den NesteEKuruvillaJWestinJ. Outcomes in Refractory Diffuse Large B-Cell Lymphoma: Results From the International SCHOLAR-1 Study. Blood (2017) 130(16):1800–8. 10.1182/blood-2017-03-769620 PMC564955028774879

[4] GisselbrechtCGlassBMounierNGillDSLinchDCTrnenyM. Salvage Regimens With Autologous Transplantation for Relapsed Large B-Cell Lymphoma in the Rituximab Era. J Clin Oncol (2010) 28(27):4184. 10.1200/JCO.2010.28.1618 20660832PMC3664033

[5] MounierNCanalsCGisselbrechtCCornelissenJFoaRCondeE. High-Dose Therapy and Autologous Stem Cell Transplantation in First Relapse for Diffuse Large B Cell Lymphoma in the Rituximab Era: An Analysis Based on Data From the European Blood and Marrow Transplantation Registry. Biol Blood Marrow Transplant (2012) 18(5):788–93. 10.1016/j.bbmt.2011.10.010 22005647

[6] LullaPDHillLCRamosCAHeslopHE. The Use of Chimeric Antigen Receptor T Cells in Patients With Non-Hodgkin Lymphoma. Clin Adv Hematol Oncol: H&O (2018) 16(5):375.29851933PMC6469642

[7] AvanziMPBrentjensRJ. Emerging Role of CAR T Cells in Non-Hodgkin’s Lymphoma. J Natl Compr Cancer Netw (2017) 15(11):1429–37. 10.6004/jnccn.2017.7045 29118234

[8] SrivastavaSRiddellSR. Engineering CAR-T Cells: Design Concepts. Trends Immunol (2015) 36(8):494–502. 10.1016/j.it.2015.06.004 26169254PMC4746114

[9] JohnsonLAJuneCH. Driving Gene-Engineered T Cell Immunotherapy of Cancer. Cell Res (2017) 27(1):38–58. 10.1038/cr.2016.154 28025979PMC5223234

[10] SadelainMBrentjensRRivièreI. The Basic Principles of Chimeric Antigen Receptor Design. Cancer Discov (2013) 3(4):388–98. 10.1158/2159-8290.CD-12-0548 PMC366758623550147

[11] SwerdlowSHCampoEPileriSAHarrisNLSteinHSiebertR. The 2016 Revision of the World Health Organization Classification of Lymphoid Neoplasms. Blood (2016) 127(20):2375–90. 10.1182/blood-2016-01-643569 PMC487422026980727

[12] ProjectIT-CL. International Peripheral T-cell and Natural Killer/T-Cell Lymphoma Study: Pathology Findings and Clinical Outcomes. J Clin Oncol (2008) 26(25):4124–30. 10.1200/JCO.2008.16.4558 18626005

[13] AbramsonJFeldmanTKroll-DesrosiersAMufflyLWinerEFlowersC. Peripheral T-Cell Lymphomas in a Large US Multicenter Cohort: Prognostication in the Modern Era Including Impact of Frontline Therapy. Ann Oncol (2014) 25(11):2211–7. 10.1093/annonc/mdu443 PMC448154325193992

[14] LeslieLASkarbnikAPBejotCStivesSFeldmanTAGoyAH. Targeting Indolent Non-Hodgkin Lymphoma. Expert Rev Hematol (2017) 10(4):299–313. 10.1080/17474086.2017.1303374 28277849

[15] McLaughlinPGrillo-LópezAJLinkBKLevyRCzuczmanMSWilliamsME. Rituximab Chimeric Anti-CD20 Monoclonal Antibody Therapy for Relapsed Indolent Lymphoma: Half of Patients Respond to a Four-Dose Treatment Program. J Clin Oncol (1998) 16(8):2825–33. 10.1200/JCO.1998.16.8.2825 9704735

[16] CoiffierBHaiounCKettererNEngertAATillyHMaD. Rituximab (anti-CD20 Monoclonal Antibody) for the Treatment of Patients With Relapsing or Refractory Aggressive Lymphoma: A Multicenter Phase II Study. Blood J Am Soc Hematol (1998) 92(6):1927–32.9731049

[17] LeungS-OGoldenbergDMDionASPellegriniMCShevitzJShihLB. Construction and Characterization of a Humanized, Internalizing, B-Cell (CD22)-Specific, Leukemia/Lymphoma Antibody, LL2. Mol Immunol (1995) 32(17-18):1413–27. 10.1016/0161-5890(95)00080-1 8643111

[18] JuweidMEStadtmauerEHajjarGSharkeyRMSuleimanSLugerS. Pharmacokinetics, Dosimetry, and Initial Therapeutic Results With 131I-and 111In-90Y-Labeled Humanized Ll2 Anti-CD22 Monoclonal Antibody in Patients With Relapsed, Refractory Non-Hodgkin’s Lymphoma. Clin Cancer Res (1999) 5(10):3292s–303s.10541378

[19] LeonardJPColemanMKetasJCChadburnAFurmanRSchusterMW. Epratuzumab, A Humanized Anti-CD22 Antibody, In Aggressive Non-Hodgkin’s Lymphoma: Phase I/II Clinical Trial Results. Clin Cancer Res (2004) 10(16):5327–34. 10.1158/1078-0432.CCR-04-0294 15328168

[20] HariharanHBerquistLMurphyTHannaNBraslawskyGLeighB. Therapeutic Application of An Anti-CD80 Antibody (IDEC-114) in B-Cell Lymphoma. J Immunother (2002) 25:S31. 10.1158/1535-7163

[21] HariharanKBerquistLMurphyTBraslawskyGHannaNLeighB. Anti-CD80 ANTIBODY (Idec-114) THERAPY for Non-Hodgkin’s Lymphoma. Ann Oncol (2002) 13:S31.

[22] VinjamaramSCzuczmanMSHernandez-IlizaliturriFJ. The Use of Galiximab in Non-Hodgkin Lymphoma. Clin Lymphoma Myeloma (2008) 8(5):277–82. 10.3816/CLM.2008.n.038 18854281

[23] MakitaSTobinaiK. Antibody Therapy Targeting CD19 for B-Cell Non-Hodgkin’s Lymphoma. >Oxford, England>: Oxford University Press (2018).10.1093/annonc/mdy09229554220

[24] AwanFTLapalombellaRTrottaRButcharJPYuBBensonDM. CD19 Targeting of Chronic Lymphocytic Leukemia With a Novel Fc-Domain–Engineered Monoclonal Antibody. Blood (2010) 115(6):1204–13. 10.1182/blood-2009-06-229039 PMC282623219965644

[25] HortonHMBernettMJPongEPeippMKarkiSChuSY. Potent *In Vitro* and *In Vivo* Activity of An Fc-engineered Anti-CD19 Monoclonal Antibody Against Lymphoma and Leukemia. Cancer Res (2008) 68(19):8049–57. 10.1158/0008-5472.CAN-08-2268 18829563

[26] LapalombellaRYehY-YWangLRamanunniARafiqSJhaS. Tetraspanin CD37 Directly Mediates Transduction of Survival and Apoptotic Signals. Cancer Cell (2012) 21(5):694–708. 10.1016/j.ccr.2012.03.040 22624718PMC3360882

[27] ZhaoXLapalombellaRJoshiTCheneyCGowdaAHayden-LedbetterMS. Targeting CD37-positive Lymphoid Malignancies With a Novel Engineered Small Modular Immunopharmaceutical. Blood J Am Soc Hematol (2007) 110(7):2569–77. 10.1182/blood-2006-12-062927 PMC198892217440052

[28] JilaniIO’BrienSManshuriTThomasDAThomazyVAImamM. Transient Down-Modulation of CD20 by Rituximab in Patients With Chronic Lymphocytic Leukemia. Blood (2003) 102(10):3514–20. 10.1182/blood-2003-01-0055 12893761

[29] KennedyADSolgaMDSchumanTAChiAWLindorferMASutherlandWM. An anti-C3b (I) mAb Enhances Complement Activation, C3b (I) Deposition, and Killing of CD20+ Cells by Rituximab. Blood J Am Soc Hematol (2003) 101(3):1071–9. 10.1182/blood-2002-03-0876 12393727

[30] WardEMitterederNKutaESimsGPBowenMADall’AcquaW. A Glycoengineered anti-CD19 Antibody With Potent Antibody-Dependent Cellular Cytotoxicity Activity *In Vitro* and Lymphoma Growth Inhibition *In Vivo* . Br J Haematol (2011) 155(4):426–37. 10.1111/j.1365-2141.2011.08857.x 21902688

[31] Forero-TorresAHamadaniMFanaleMABelloCMKippsTJOffnerF. Safety Profile and Clinical Response to MEDI-551, A Humanized Monoclonal Anti-CD19, in a Phase 1/2 Study in Adults With Relapsed or Refractory Advanced B-Cell Malignancies. Am Soc Hematol Washington DC (2013) 122. 10.1182/blood.V120.21.3677.3677

[32] PolsonAGYuS-FElkinsKZhengBClarkSIngleGS. Antibody-Drug Conjugates Targeted to CD79 for the Treatment of Non-Hodgkin Lymphoma. Blood (2007) 110(2):616–23. 10.1182/blood-2007-01-066704 17374736

[33] ChuY-WPolsonA. Antibody–Drug Conjugates for the Treatment of B-Cell Non-Hodgkin’s Lymphoma and Leukemia. Future Oncol (2013) 9(3):355–68. 10.2217/fon.12.189 23469971

[34] LuTGibianskyLLiXLiCShiRAgarwalP. Exposure-Safety and Exposure-Efficacy Analyses of Polatuzumab Vedotin in Patients With Relapsed or Refractory Diffuse Large B-Cell Lymphoma. Leuk Lymphoma (2020) 61(12):2905–14. 10.1080/10428194.2020.1795154 32705923

[35] HarrisLJPatelKMartinM. Novel Therapies for Relapsed or Refractory Diffuse Large B-Cell Lymphoma. Int J Mol Sci (2020) 21(22):8553. 10.3390/ijms21228553 PMC769811733202794

[36] FanaleMAForero-TorresARosenblattJDAdvaniRHFranklinARKennedyDA. A Phase I Weekly Dosing Study of Brentuximab Vedotin in Patients With Relapsed/Refractory CD30-Positive Hematologic Malignancies. Clin Cancer Res (2012) 18(1):248–55. 10.1158/1078-0432.CCR-11-1425 22080439

[37] FranciscoJACervenyCGMeyerDLMixanBJKlussmanKChaceDF. cAC10-vcMMAE, An Anti-CD30–Monomethyl Auristatin E Conjugate With Potent and Selective Antitumor Activity. Blood (2003) 102(4):1458–65. 10.1182/blood-2003-01-0039 12714494

[38] JacobsenEDSharmanJPOkiYAdvaniRHWinterJNBelloCM. Brentuximab Vedotin Demonstrates Objective Responses in a Phase 2 Study of Relapsed/Refractory DLBCL With Variable CD30 Expression. Blood J Am Soc Hematol (2015) 125(9):1394–402. 10.1182/blood-2014-09-598763 25573987

[39] LensSMDrillenburgPDen DrijverBFVan SchijndelGPalsSTVan LierRA. Aberrant Expression and Reverse Signalling of CD70 on Malignant B Cells. Br J Haematol (1999) 106(2):491–503. 10.1046/j.1365-2141.1999.01573.x 10460611

[40] DoroninaSOMendelsohnBABoveeTDCervenyCGAlleySCMeyerDL. Enhanced Activity of Monomethylauristatin F Through Monoclonal Antibody Delivery: Effects of Linker Technology on Efficacy and Toxicity. Bioconjugate Chem (2006) 17(1):114–24. 10.1021/bc0502917 16417259

[41] AlleySCBenjaminDRJeffreySCOkeleyNMMeyerDLSandersonRJ. Contribution of Linker Stability to the Activities of Anticancer Immunoconjugates. Bioconjugate Chem (2008) 19(3):759–65. 10.1021/bc7004329 18314937

[42] ShorBGerberH-PSapraP. Preclinical and Clinical Development of Inotuzumab-Ozogamicin in Hematological Malignancies. Mol Immunol (2015) 67(2):107–16. 10.1016/j.molimm.2014.09.014 25304309

[43] YurkiewiczIRMufflyLLiedtkeM. Inotuzumab Ozogamicin: A CD22 mAb–Drug Conjugate for Adult Relapsed or Refractory B-Cell Precursor Acute Lymphoblastic Leukemia. Drug Des Dev Ther (2018) 12:2293. 10.2147/DDDT.S150317 PMC606324630087554

[44] RaufiAEbrahimASAl-KatibA. Targeting CD19 in B-Cell Lymphoma: Emerging Role of SAR3419. Cancer Manage Res (2013) 5:225. 10.2147/CMAR.S45957 PMC376748724023523

[45] PressOWEaryJFBadgerCCMartinPJAppelbaumFRLevyR. Treatment of Refractory Non-Hodgkin’s Lymphoma With Radiolabeled MB-1 (Anti-CD37) Antibody. J Clin Oncol (1989) 7(8):1027–38. 10.1200/JCO.1989.7.8.1027 2666588

[46] DeckertJParkPUChicklasSYiYLiMLaiKC. A Novel anti-CD37 Antibody-Drug Conjugate With Multiple Anti-Tumor Mechanisms for the Treatment of B-Cell Malignancies. Blood (2013) 122(20):3500–10. The Journal of the American Society of Hematology. 10.1182/blood-2013-05-505685 24002446

[47] AlinariLQuinionCBlumKA. Bruton’s Tyrosine Kinase Inhibitors in B-Cell Non-Hodgkin’s Lymphomas. Clin Pharmacol Ther (2015) 97(5):469–77. 10.1002/cpt.65 25670208

[48] AalipourAAdvaniRH. Bruton’s Tyrosine Kinase Inhibitors and Their Clinical Potential in the Treatment of B-Cell Malignancies: Focus on Ibrutinib. Ther Adv Hematol (2014) 5(4):121–33. 10.1177/2040620714539906 PMC421231325360238

[49] HerreraAFGoyAMehtaARamchandrenRPagelJMSvobodaJ. Safety and Activity of Ibrutinib in Combination With Durvalumab in Patients With Relapsed or Refractory Follicular Lymphoma or Diffuse Large B-Cell Lymphoma. Am J Hematol (2020) 95(1):18–27. 10.1002/ajh.25659 31621094PMC6904508

[50] DubovskyJABeckwithKANatarajanGWoyachJAJaglowskiSZhongY. Ibrutinib is an Irreversible Molecular Inhibitor of ITK Driving a Th1-Selective Pressure in T Lymphocytes. Blood (2013) 122(15):2539–49. 10.1182/blood-2013-06-507947 PMC379545723886836

[51] CoveyTBarfTGulrajaniMKrantzFvan LithBBibikovaE. Acp-196: A Novel Covalent Bruton’s Tyrosine Kinase (Btk) Inhibitor With Improved Selectivity and *In Vivo* Target Coverage in Chronic Lymphocytic Leukemia (CLL) Patients. AACR (2015). 10.1158/1538-7445.AM2015-2596

[52] ByrdJCHarringtonBO’BrienSJonesJASchuhADevereuxS. Acalabrutinib (ACP-196) in Relapsed Chronic Lymphocytic Leukemia. New Engl J Med (2016) 374(4):323–32. 10.1056/NEJMoa1509981 PMC486258626641137

[53] ThorpeLMYuzugulluHZhaoJJ. PI3K in Cancer: Divergent Roles of Isoforms, Modes of Activation and Therapeutic Targeting. Nat Rev Cancer (2015) 15(1):7–24. 10.1038/nrc3860 25533673PMC4384662

[54] VanhaesebroeckBWelhamMJKotaniKSteinRWarnePHZvelebilMJ. P110δ, A Novel Phosphoinositide 3-Kinase in Leukocytes. Proc Natl Acad Sci (1997) 94(9):4330–5. 10.1073/pnas.94.9.4330 PMC207229113989

[55] SamuelsYWangZBardelliASillimanNPtakJSzaboS. High Frequency of Mutations of the PIK3CA Gene in Human Cancers. Science (2004) 304:554. 10.1126/science.1096502 15016963

[56] PaulJSoujonMWengnerAMZitzmann-KolbeSSturzAHaikeK. Simultaneous Inhibition of PI3Kδ and PI3Kα Induces ABC-DLBCL Regression by Blocking BCR-dependent and-Independent Activation of NF-κb and AKT. Cancer Cell (2017) 31(1):64–78. 10.1016/j.ccell.2016.12.003 28073005

[57] IyengarSClearABödörCMaharajLLeeACalaminiciM. P110α-Mediated Constitutive PI3K Signaling Limits the Efficacy of P110δ-Selective Inhibition in Mantle Cell Lymphoma, Particularly With Multiple Relapse. Blood (2013) 121(12):2274–84. The Journal of the American Society of Hematology. 10.1182/blood-2012-10-460832 PMC360606423341541

[58] ErdmannTKlenerPLynchJTGrauMVočkováPMolinskyJ. Sensitivity to PI3K and AKT Inhibitors is Mediated by Divergent Molecular Mechanisms in Subtypes of DLBCL. Blood (2017) 130(3):310–22. 10.1182/blood-2016-12-758599 28202458

[59] NarkhedeMChesonBD. Copanlisib in the Treatment of Non-Hodgkin Lymphoma. Future Oncol (2020) 16(26):1947–55. 10.2217/fon-2020-0195 32658557

[60] PaiettaE. Immunobiology of Acute Leukemia. Neoplastic Dis Blood: Springer; (2018) p:237–79. 10.1007/978-3-319-64263-5_15

[61] BalakrishnanKPelusoMFuMRosinNBurgerJAWierdaWG. The phosphoinositide-3-kinase (PI3K)-Delta and Gamma Inhibitor, IPI-145 (Duvelisib), Overcomes Signals From the PI3K/AKT/S6 Pathway and Promotes Apoptosis in CLL. Leukemia (2015) 29(9):1811–22. 10.1038/leu.2015.105 PMC455837425917267

[62] AliAYWuXEissaNHouSGhiaJ-EMurookaTT. Distinct Roles for Phosphoinositide 3-Kinases γ and δ in Malignant B Cell Migration. Leukemia (2018) 32(9):1958–69. 10.1038/s41375-018-0012-5 PMC612708729479062

[63] GrafSAGopalAK. Idelalisib for the Treatment of Non-Hodgkin Lymphoma. Expert Opin Pharmacother (2016) 17(2):265–74. 10.1517/14656566.2016.1135130 PMC495580526818003

[64] CornallRJChengAMPawsonTGoodnowCC. Role of Syk in B-Cell Development and Antigen-Receptor Signaling. Proc Natl Acad Sci (2000) 97(4):1713–8. 10.1073/pnas.97.4.1713 PMC2650110677523

[65] ChengSCoffeyGZhangXHShaknovichRSongZLuP. SYK Inhibition and Response Prediction in Diffuse Large B-Cell Lymphoma. Blood J Am Soc Hematol (2011) 118(24):6342–52. 10.1182/blood-2011-02-333773 22025527

[66] GururajanMJenningsCDBondadaS. Cutting Edge: Constitutive B Cell Receptor Signaling Is Critical for Basal Growth of B Lymphoma. J Immunol (2006) 176(10):5715–9. 10.4049/jimmunol.176.10.5715 16670274

[67] BuchnerMFuchsSPrinzGPfeiferDBartholoméKBurgerM. Spleen Tyrosine Kinase Is Overexpressed and Represents a Potential Therapeutic Target in Chronic Lymphocytic Leukemia. Cancer Res (2009) 69(13):5424–32. 10.1158/0008-5472.CAN-08-4252 19549911

[68] AndorskyDJKolibabaKSAssoulineSForero-TorresAJonesVKleinLM. An Open-Label Phase 2 Trial of Entospletinib in Indolent Non-Hodgkin Lymphoma and Mantle Cell Lymphoma. Br J Haematol (2019) 184(2):215–22. 10.1111/bjh.15552 PMC658596030183069

[69] BraselmannSTaylorVZhaoHWangSSylvainCBaluomM. R406, An Orally Available Spleen Tyrosine Kinase Inhibitor Blocks Fc Receptor Signaling and Reduces Immune Complex-Mediated Inflammation. J Pharmacol Exp Ther (2006) 319(3):998–1008. 10.1124/jpet.106.109058 16946104

[70] WeinblattMEKavanaughABurgos-VargasRDikranianAHMedrano-RamirezGMorales-TorresJL. Treatment of Rheumatoid Arthritis With a Syk Kinase Inhibitor: A Twelve-Week, Randomized, Placebo-Controlled Trial. Arthritis Rheum (2008) 58(11):3309–18. 10.1002/art.23992 18975322

[71] PodolanczukALazarusAHCrowARGrossbardEBusselJB. Of Mice and Men: An Open-Label Pilot Study for Treatment of Immune Thrombocytopenic Purpura by An Inhibitor of Syk. Blood (2009) 113(14):3154–60. 10.1182/blood-2008-07-166439 19096013

[72] RobertsAW. Therapeutic Development and Current Uses of BCL-2 Inhibition. In: Hematology 2014, the American Society of Hematology Education Program Book, vol. 2020. ASH (2020). p. 1–9.10.1182/hematology.2020000154PMC772756933275682

[73] SekiguchiNKobayashiYYokotaYKusumotoSTanimotoKWatanabeT. Follicular Lymphoma Subgrouping by Fluorescence *In Situ* Hybridization Analysis. Cancer Sci (2005) 96(2):77–82. 10.1111/j.1349-7006.2005.00014.x 15723651PMC11159974

[74] TsujimotoYFingerLRYunisJNowellPCCroceCM. Cloning of the Chromosome Breakpoint of Neoplastic B Cells With the T (14; 18) Chromosome Translocation. Science (1984) 226(4678):1097–9. 10.1126/science.6093263 6093263

[75] WeiMC. Bcl-2-related Genes in Lymphoid Neoplasia. Int J Hematol (2004) 80(3):205–9. 10.1532/IJH97.04110 15540893

[76] TseCShoemakerARAdickesJAndersonMGChenJJinS. Abt-263: A Potent and Orally Bioavailable Bcl-2 Family Inhibitor. Cancer Res (2008) 68(9):3421–8. 10.1158/0008-5472.CAN-07-5836 18451170

[77] LockRCarolHHoughtonPJMortonCLKolbEAGorlickR. Initial Testing (Stage 1) of the BH3 Mimetic ABT-263 by the Pediatric Preclinical Testing Program. Pediatr Blood Cancer (2008) 50(6):1181–9. 10.1002/pbc.21433 18085673

[78] MasonKKhawSRayerouxKChewELeeEFairlieW. The BH3 Mimetic Compound, ABT-737, Synergizes With a Range of Cytotoxic Chemotherapy Agents in Chronic Lymphocytic Leukemia. Leukemia (2009) 23(11):2034–41. 10.1038/leu.2009.151 19641525

[79] WangYCastanarRBolosJ. Abt-263. Drugs Fut (2008) 33:829–37. 10.1358/dof.2008.33.10.1265203

[80] DavidsMSRobertsAWSeymourJFPagelJMKahlBSWierdaWG. Phase I First-in-Human Study of Venetoclax in Patients With Relapsed or Refractory non-Hodgkin Lymphoma. J Clin Oncol (2017) 35(8):826. 10.1200/JCO.2016.70.4320 28095146PMC5455685

[81] FranciscoLMSagePTSharpeAH. The PD-1 Pathway in Tolerance and Autoimmunity. Immunol Rev (2010) 236(1):219–42. 10.1111/j.1600-065X.2010.00923.x PMC291927520636820

[82] PardollDM. The Blockade of Immune Checkpoints in Cancer Immunotherapy. Nat Rev Cancer (2012) 12(4):252–64. 10.1038/nrc3239 PMC485602322437870

[83] HuiECheungJZhuJSuXTaylorMJWallweberHA. T Cell Costimulatory Receptor CD28 is a Primary Target for PD-1–mediated Inhibition. Science (2017) 355(6332):1428–33. 10.1126/science.aaf1292 PMC628607728280247

[84] AndorskyDJYamadaRESaidJPinkusGSBettingDJTimmermanJM. Programmed Death Ligand 1 is Expressed by Non–Hodgkin Lymphomas and Inhibits the Activity of Tumor-Associated T Cells. Clin Cancer Res (2011) 17(13):4232–44. 10.1158/1078-0432.CCR-10-2660 21540239

[85] KiyasuJMiyoshiHHirataAArakawaFIchikawaANiinoD. Expression of Programmed Cell Death Ligand 1 Is Associated With Poor Overall Survival in Patients With Diffuse Large B-Cell Lymphoma. Blood (2015) 126(19):2193–201. 10.1182/blood-2015-02-629600 PMC463511526239088

[86] CarrerasJLopez-GuillermoARoncadorGVillamorNColomoLMartinezA. High Numbers of Tumor-Infiltrating Programmed Cell Death 1–Positive Regulatory Lymphocytes Are Associated With Improved Overall Survival in Follicular Lymphoma. J Clin Oncol (2009) 27(9):1470–6. 10.1200/JCO.2008.18.0513 19224853

[87] GongJChehrazi-RaffleAReddiSSalgiaR. Development of PD-1 and PD-L1 Inhibitors as a Form of Cancer Immunotherapy: A Comprehensive Review of Registration Trials and Future Considerations. J Immunother Cancer (2018) 6(1):8. 10.1186/s40425-018-0316-z 29357948PMC5778665

[88] IbrahimRStewartRShalabiA. Pd-L1 Blockade for Cancer Treatment: MEDI4736. Semin Oncol (2015) 42:474-83. Elsevier. 10.1053/j.seminoncol.2015.02.007 25965366

[89] Sagiv-BarfiIKohrtHECzerwinskiDKNgPPChangBYLevyR. Therapeutic Antitumor Immunity by Checkpoint Blockade is Enhanced by Ibrutinib, An Inhibitor of Both BTK and ITK. Proc Natl Acad Sci (2015) 112(9):E966–E72. 10.1073/pnas.1500712112 PMC435277725730880

[90] ArmandPJanssensAMGrittiGRadfordJTimmermanJMPintoA. Efficacy and Safety Results From CheckMate 140, A Phase 2 Study of Nivolumab for Relapsed/Refractory Follicular Lymphoma. Blood (2020) 137:637–45. 10.1182/blood.2019004753 PMC786918832870269

[91] SheikhSKuruvillaJ. Pembrolizumab for the Treatment of Diffuse Large B-Cell Lymphoma. Expert Opin Biol Ther (2019) 19(11):1119–26. 10.1080/14712598.2019.1659777 31456438

[92] TwaDDSteidlC. Structural Genomic Alterations in Primary Mediastinal Large B-Cell Lymphoma. Leuk Lymphoma (2015) 56(8):2239–50. 10.3109/10428194.2014.985673 25393674

[93] MerrymanRWArmandPWrightKTRodigSJ. Checkpoint Blockade in Hodgkin and Non-Hodgkin Lymphoma. Blood Adv (2017) 1(26):2643–54. 10.1182/bloodadvances.2017012534 PMC572864629296917

[94] HudeISasseSEngertABröckelmannPJ. The Emerging Role of Immune Checkpoint Inhibition in Malignant Lymphoma. Haematologica (2017) 102(1):30–42. 10.3324/haematol.2016.150656 27884973PMC5210230

[95] IshidaYAgataYShibaharaKHonjoT. Induced Expression of PD-1, a Novel Member of the Immunoglobulin Gene Superfamily, Upon Programmed Cell Death. EMBO J (1992) 11(11):3887–95. 10.1002/j.1460-2075.1992.tb05481.x PMC5568981396582

[96] KeirMEButteMJFreemanGJSharpeAH. PD-1 and its Ligands in Tolerance and Immunity. Annu Rev Immunol (2008) 26:677–704. 10.1146/annurev.immunol.26.021607.090331 18173375PMC10637733

[97] QuezadaSPeggsK. Exploiting CTLA-4, PD-1 and PD-L1 to Reactivate the Host Immune Response Against Cancer. Br J Cancer (2013) 108(8):1560–5. 10.1038/bjc.2013.117 PMC366848323511566

[98] JacobsenED. Restoring Antitumor Immunity *Via* PD-1 Blockade After Autologous Stem-Cell Transplantation for Diffuse Large B-Cell Lymphoma. J Clin Oncol (2013) 31(33):4268–70. 10.1200/JCO.2013.51.7680 24127445

[99] BryanLJGordonLI. Pidilizumab in the Treatment of Diffuse Large B-Cell Lymphoma. Expert Opin Biol Ther (2014) 14(9):1361–8. 10.1517/14712598.2014.942637 25056108

[100] ChowKUSommerladWDBoehrerSSchneiderBSeipeltGRummelMJ. Anti-CD20 Antibody (IDEC-C2B8, Rituximab) Enhances Efficacy of Cytotoxic Drugs on Neoplastic Lymphocytes *In Vitro*: Role of Cytokines, Complement, and Caspases. haematologica (2002) 87(1):33–43.11801463

[101] KanekalSCrainBElliottG. Sdx-105 (Treanda™) Enhances the Tumor Growth Inhibitory Effect of Rituximab in Daudi Lymphoma Xenografts. Am Soc Hematol (2004). 21:266 10.1182/blood.V104.11.4580.4580

[102] Garnock-JonesKP. Bendamustine. Drugs (2010) 70(13):1703–18. 10.2165/11205860-000000000-00000 20731477

[103] Leonard J Epratuzumab (Anti-CD22) and Rituximab (Anti-CD20) Combination Immunotherapy for Non-Hodgkin’s Lymphoma: Preliminary Response Data. Proc Am Soc Clin Oncol (2001) 120:361–70.

[104] SallesGADuellJGonzález-BarcaEJurczakWLiberatiAMNagyZ. Single-Arm Phase II Study of MOR208 Combined With Lenalidomide in Patients With Relapsed or Refractory Diffuse Large B-Cell Lymphoma: L-Mind. Blood (2017) 130(Supplement 1):4123–. 10.1182/blood-2018-99-113399

[105] AlgatePAWiensJNilssonCShoMChaoDTStarlingGC. Tru-016, An Anti-Cd37 SMIP™ Biologic, In Combination With Other Therapeutic Drugs in Models of non-Hodgkin’s Lymphoma. Am Soc Hematol (2010). 10.1182/blood.V116.21.3931.3931

[106] Wagner-JohnstonNGoyARodriguezMAEhmannCHamlinPRadfordJ. Anti-CD22 Immunoconjugate Inotuzumab Ozogamicin+ Rituximab Followed by Stem Cell Transplantation in Relapsed/Refractory DLBCL Patients: Safety and Efficacy. Am Soc Hematol (2011) 2718. 10.1182/blood.V118.21.2718.2718

[107] DangNHSmithMROffnerFVerhoefGJohnsonPRohatinerAZ. Anti-CD22 Immunoconjugate Inotuzumab Ozogamicin (Cmc-544)+ Rituximab: Clinical Activity Including Survival in Patients With Recurrent/Refractory Follicular or ‘Aggressive’lymphoma. Am Soc Hematol (2009) 114:242–3. 10.1182/blood.V114.22.584.584

[108] OguraMUchidaTMacDonaldDAHatakeKDaviesASanghaR. An Open-Label, Phase I Study of R-CVP in Combination With Inotuzumab Ozogamicin in Patients With Relapsed/Refractory CD22-positive B-Cell Non-Hodgkin Lymphoma. Am Soc Hematol (2011) 118. 10.1182/blood.V118.21.3715.3715

[109] SahakianERock-KlotzJShahBDPowersJCultreraJLDengS. Combination of ACY1215, a Selective Histone Deacetylase 6 (HDAC6) Inhibitor With the Bruton Tyrosine Kinase (BTK) Inhibitor, Ibrutinib, Represents a Novel Therapeutic Strategy in Mantle Cell Lymphoma (MCL). Am Soc Hematol (2012), 1660. 10.1182/blood.V120.21.1660.1660

[110] DasmahapatraGPatelHDentPFisherRIFriedbergJGrantS. The Bruton Tyrosine Kinase (BTK) Inhibitor PCI-32765 Synergistically Increases Proteasome Inhibitor Activity in Diffuse Large-B Cell Lymphoma (DLBCL) and Mantle Cell Lymphoma (MCL) Cells Sensitive or Resistant to Bortezomib. Br J Haematol (2013) 161(1):43–56. 10.1111/bjh.12206 23360303PMC3739300

[111] YangYShafferALIIIEmreNTCeribelliMZhangMWrightG. Exploiting Synthetic Lethality for the Therapy of ABC Diffuse Large B Cell Lymphoma. Cancer Cell (2012) 21(6):723–37. 10.1016/j.ccr.2012.05.024 PMC405983322698399

[112] de RooijMFKuilAKaterAPKerstenMJPalsSTSpaargarenM. Ibrutinib and Idelalisib Synergistically Target BCR-Controlled Adhesion in MCL and CLL: A Rationale for Combination Therapy. Blood J Am Soc Hematol (2015) 125(14):2306–9. 10.1182/blood-2014-12-619163 PMC441694025838279

[113] RobertsAWAdvaniRHKahlBSPerskyDSweetenhamJWCarneyDA. Phase 1 Study of the Safety, Pharmacokinetics, and Antitumour Activity of the BCL 2 Inhibitor Navitoclax in Combination With Rituximab in Patients With Relapsed or Refractory CD 20+ Lymphoid Malignancies. Br J Haematol (2015) 170(5):669–78. 10.1111/bjh.13487 PMC453431425942994

[114] KippsTJEradatHGrosickiSCatalanoJCosoloWDyagilIS. A Phase 2 Study of the BH3 Mimetic BCL2 Inhibitor Navitoclax (ABT-263) With or Without Rituximab, In Previously Untreated B-Cell Chronic Lymphocytic Leukemia. Leuk Lymphoma (2015) 56(10):2826–33. 10.3109/10428194.2015.1030638 PMC464341725797560

[115] AcklerSMittenMChenJClarinJFosterKJinS. Navitoclax (ABT-263) and Bendamustine±Rituximab Induce Enhanced Killing of Non-Hodgkin’s Lymphoma Tumours *In Vivo* . Br J Pharmacol (2012) 167(4):881–91. 10.1111/j.1476-5381.2012.02048.x PMC357578622624727

[116] PhamLVHuangSZhangHZhangJBellTZhouS. Strategic Therapeutic Targeting to Overcome Venetoclax Resistance in Aggressive B-Cell Lymphomas. Clin Cancer Res (2018) 24(16):3967–80. 10.1158/1078-0432.CCR-17-3004 29666304

[117] LiLPongtornpipatPTiutanTKendrickSLParkSPerskyDO. Synergistic Induction of Apoptosis in High-Risk DLBCL by BCL2 Inhibition With ABT-199 Combined With Pharmacologic Loss of MCL1. Leukemia (2015) 29(8):1702–12. 10.1038/leu.2015.99 PMC452634325882699

[118] de VosSSwinnenLWangDReidEFowlerNCorderoJ. Venetoclax, Bendamustine, and Rituximab in Patients With Relapsed or Refractory NHL: A Phase Ib Dose-Finding Study. Ann Oncol (2018) 29(9):1932–8. 10.1093/annonc/mdy256 PMC615876230060083

[119] TamCSAndersonMAPottCAgarwalRHandunnettiSHicksRJ. Ibrutinib Plus Venetoclax for the Treatment of Mantle-Cell Lymphoma. New Engl J Med (2018) 378(13):1211–23. 10.1056/NEJMoa1715519 29590547

[120] WangXRivièreI. Clinical Manufacturing of CAR T Cells: Foundation of a Promising Therapy. Mol Ther-Oncol (2016) 3:16015. 10.1038/mto.2016.15 PMC490909527347557

[121] FenskeTSAhnKWGraffTMDiGilioABashirQKambleRT. Allogeneic Transplantation Provides Durable Remission in a Subset of DLBCL Patients Relapsing After Autologous Transplantation. Br J Haematol (2016) 174(2):235–48. 10.1111/bjh.14046 PMC494028226989808

[122] PastoreAJurinovicVKridelRHosterEStaigerAMSzczepanowskiM. Integration of Gene Mutations in Risk Prognostication for Patients Receiving First-Line Immunochemotherapy for Follicular Lymphoma: A Retrospective Analysis of a Prospective Clinical Trial and Validation in a Population-Based Registry. Lancet Oncol (2015) 16(9):1111–22. 10.1016/S1470-2045(15)00169-2 26256760

[123] BarrettDMGruppSAJuneCH. Chimeric Antigen Receptor–and TCR-Modified T Cells Enter Main Street and Wall Street. J Immunol (2015) 195(3):755–61. 10.4049/jimmunol.1500751 PMC450728626188068

[124] HudecekMSommermeyerDKosasihPLSilva-BenedictALiuLRaderC. The Nonsignaling Extracellular Spacer Domain of Chimeric Antigen Receptors is Decisive for In Vivo Antitumor Activity. Cancer Immunol Res (2015) 3(2):125–35. 10.1158/2326-6066.CIR-14-0127 PMC469280125212991

[125] ZhaoZCondominesMvan der StegenSJPernaFKlossCCGunsetG. Structural Design of Engineered Costimulation Determines Tumor Rejection Kinetics and Persistence of CAR T Cells. Cancer Cell (2015) 28(4):415–28. 10.1016/j.ccell.2015.09.004 PMC500305626461090

[126] LouisCUSavoldoBDottiGPuleMYvonEMyersGD. Antitumor Activity and Long-Term Fate of Chimeric Antigen Receptor–Positive T Cells in Patients With Neuroblastoma. Blood (2011) 118(23):6050–6. The Journal of the American Society of Hematology. 10.1182/blood-2011-05-354449 PMC323466421984804

[127] SadelainM. CAR Therapy: The CD19 Paradigm. J Clin Invest (2015) 125(9):3392–400. 10.1172/JCI80010 PMC458828126325036

[128] EshharZ. The T-body Approach: Redirecting T Cells With Antibody Specificity. In: Therapeutic Antibodies. New York, USA: Springer (2008). p. 329–42.10.1007/978-3-540-73259-4_1418071952

[129] TillBGJensenMCWangJQianXGopalAKMaloneyDG. CD20-Specific Adoptive Immunotherapy for Lymphoma Using a Chimeric Antigen Receptor With Both CD28 and 4-1BB Domains: Pilot Clinical Trial Results. Blood (2012) 119(17):3940–50. The Journal of the American Society of Hematology. 10.1182/blood-2011-10-387969 PMC335036122308288

[130] BrentjensRYehRBernalYRiviereISadelainM. Treatment of Chronic Lymphocytic Leukemia With Genetically Targeted Autologous T Cells: Case Report of An Unforeseen Adverse Event in a Phase I Clinical Trial. Mol Ther (2010) 18(4):666–8. 10.1038/mt.2010.31 PMC286252520357779

[131] ParkJHBrentjensRJ. Are All Chimeric Antigen Receptors Created Equal? J Clin Oncol (2015) 33(6):651–3. 10.1200/JCO.2014.57.5472 25605860

[132] QianLLiDMaLHeTQiFShenJ. The Novel anti-CD19 Chimeric Antigen Receptors With Humanized scFv (Single-Chain Variable Fragment) Trigger Leukemia Cell Killing. Cell Immunol (2016) 304:49–54. 10.1016/j.cellimm.2016.03.003 26996927

[133] LockDMockel-TenbrinckNDrechselKBarthCMauerDSchaserT. Automated Manufacturing of Potent CD20-directed Chimeric Antigen Receptor T Cells for Clinical Use. Hum Gene Ther (2017) 28(10):914–25. 10.1089/hum.2017.111 28847167

[134] KueberuwaGKalaitsidouMCheadleEHawkinsREGilhamDE. Cd19 Car T Cells Expressing IL-12 Eradicate Lymphoma in Fully Lymphoreplete Mice Through Induction of Host Immunity. Mol Ther-Oncol (2018) 8:41–51. 10.1016/j.omto.2017.12.003 PMC577201129367945

[135] ChmielewskiMAbkenH. Trucks: The Fourth Generation of Cars. Expert Opin Biol Ther (2015) 15(8):1145–54. 10.1517/14712598.2015.1046430 25985798

[136] RaponiSStefania De ProprisMIntoppaSLaura MilaniMVitaleAEliaL. Flow Cytometric Study of Potential Target Antigens (CD19, CD20, Cd22, CD33) for Antibody-Based Immunotherapy in Acute Lymphoblastic Leukemia: Analysis of 552 Cases. Leuk Lymphoma (2011) 52(6):1098–107. 10.3109/10428194.2011.559668 21348573

[137] MamonkinMRouceRHTashiroHBrennerMK. A T-Cell–Directed Chimeric Antigen Receptor for the Selective Treatment of T-Cell Malignancies. Blood J Am Soc Hematol (2015) 126(8):983–92. 10.1182/blood-2015-02-629527 PMC454323126056165

[138] KehrlJHRivaAWilsonGLThéveninC. Molecular Mechanisms Regulating CD19, CD20 and CD22 Gene Expression. Immunol Today (1994) 15(9):432–6. 10.1016/0167-5699(94)90273-9 7524520

[139] Van Der StegenSJHamiehMSadelainM. The Pharmacology of Second-Generation Chimeric Antigen Receptors. Nat Rev Drug Discovery (2015) 14(7):499–509. 10.1038/nrd4597 26129802PMC6410718

[140] JensenMCPopplewellLCooperLJDiGiustoDKalosMOstbergJR. Antitransgene Rejection Responses Contribute to Attenuated Persistence of Adoptively Transferred CD20/CD19-Specific Chimeric Antigen Receptor Redirected T Cells in Humans. Biol Blood Marrow Transplant (2010) 16(9):1245–56. 10.1016/j.bbmt.2010.03.014 PMC338380320304086

[141] BrentjensRJSantosENikhaminYYehRMatsushitaMLa PerleK. Genetically Targeted T Cells Eradicate Systemic Acute Lymphoblastic Leukemia Xenografts. Clin Cancer Res (2007) 13(18):5426–35. 10.1158/1078-0432.CCR-07-0674 17855649

[142] KochenderferJNWilsonWHJanikJEDudleyMEStetler-StevensonMFeldmanSA. Eradication of B-Lineage Cells and Regression of Lymphoma in a Patient Treated With Autologous T Cells Genetically Engineered to Recognize CD19. Blood (2010) 116(20):4099–102. 10.1182/blood-2010-04-281931 PMC299361720668228

[143] ChagantiSIllidgeTBarringtonSMckayPLintonKCwynarskiK. Guidelines for the Management of Diffuse Large B-Cell Lymphoma. Br J Haematol (2016) 174(1):43–56. 10.1111/bjh.14136 27196701

[144] ArmitageJO. How I Treat Patients With Diffuse Large B-Cell Lymphoma. Blood J Am Soc Hematol (2007) 110(1):29–36. 10.1182/blood-2007-01-041871 17360935

[145] CostaLJMaddocksKEpperlaNReddyNMKarmaliRUmyarovaE. Diffuse Large B-Cell Lymphoma With Primary Treatment Failure: Ultra-High Risk Features and Benchmarking for Experimental Therapies. Am J Hematol (2017) 92(2):161–70. 10.1002/ajh.24615 PMC554993627880984

[146] ScheuermannRRacilaE. CD19 Antigen in Leukemia and Lymphoma Diagnosis and Immunotherapy. Leuk Lymphoma (1995) 18(5-6):385–97. 10.3109/10428199509059636 8528044

[147] KochenderferJNDudleyMEKassimSHSomervilleRPCarpenterROStetler-StevensonM. Chemotherapy-Refractory Diffuse Large B-Cell Lymphoma and Indolent B-Cell Malignancies Can Be Effectively Treated With Autologous T Cells Expressing An Anti-CD19 Chimeric Antigen Receptor. J Clin Oncol (2015) 33(6):540. 10.1200/JCO.2014.56.2025 25154820PMC4322257

[148] StirrupsR. Car T-Cell Therapy in Refractory Large B-Cell Lymphoma. Lancet Oncol (2018) 19(1):e19. 10.1016/S1470-2045(17)30928-2 29249304

[149] KridelRSehnLHGascoyneRD. Pathogenesis of Follicular Lymphoma. J Clin Invest (2012) 122(10):3424–31. 10.1172/JCI63186 PMC346191423023713

[150] HiddemannWChesonB. How We Manage Follicular Lymphoma. Leukemia (2014) 28(7):1388–95. 10.1038/leu.2014.91 24577532

[151] Selection WECotMedicines UoEOrganization WH. The Selection and Use of Essential Medicines: Report of the WHO Expert Committee, 2013 (Including the 18th WHO Model List of Essential Medicines and the 4th WHO Model List of Essential Medicines for Children). World Health Organization (2014).

[152] SchusterSJSvobodaJChongEANastaSDMatoARAnakÖ. Chimeric Antigen Receptor T Cells in Refractory B-cell Lymphomas. New Engl J Med (2017) 377(26):2545–54. 10.1056/NEJMoa1708566 PMC578856629226764

[153] ChenLXuBLongXGuJLouYWangD. Car T-cell Therapy for a Relapsed/Refractory Acute B-Cell Lymphoblastic Lymphoma Patient in the Context of Li-Fraumeni Syndrome. J Immunother Cancer (2020) 8(1):e000364. 10.1136/jitc-2019-000364 32345625PMC7213909

[154] NeelapuSS. An Interim Analysis of the ZUMA-1 Study of KTE-C19 in Refractory, Aggressive Non-Hodgkin Lymphoma. Clin Adv Hematol Oncol: H&O (2017) 15(2):117–20.28398281

[155] CheahCYSeymourJFWangML. Mantle Cell Lymphoma. J Clin Oncol (2016) 34(11):1256–69. 10.1200/JCO.2015.63.5904 26755518

[156] MaddocksK. Update on Mantle Cell Lymphoma. Blood J Am Soc Hematol (2018) 132(16):1647–56. 10.1182/blood-2018-03-791392 30154113

[157] DuJZhangY. Sequential anti-CD19, 22, and 20 Autologous Chimeric Antigen Receptor T-Cell (Car-T) Treatments of a Child With Relapsed Refractory Burkitt Lymphoma: A Case Report and Literature Review. J Cancer Res Clin Oncol (2020) 146(6):1575–82. 10.1007/s00432-020-03198-7 PMC1180445832222815

[158] YanWLiuZLiuJXiaYHuKYuJ. Application of Chimeric Antigen Receptor T Cells in the Treatment of Hematological Malignancies. BioMed Res Int (2020) 2020:4241864. 10.1155/2020/4241864 PMC754733633062678

[159] BridgemanJSLadellKSheardVMinersKHawkinsRPriceD. CD 3ζ-Based Chimeric Antigen Receptors Mediate T Cell Activation *Via* Cis-and Trans-Signalling Mechanisms: Implications for Optimization of Receptor Structure for Adoptive Cell Therapy. Clin Exp Immunol (2014) 175(2):258–67. 10.1111/cei.12216 PMC389241724116999

[160] MakitaSImaizumiKKurosawaSTobinaiK. Chimeric Antigen Receptor T-cell Therapy for B-Cell Non-Hodgkin Lymphoma: Opportunities and Challenges. Drugs Context (2019) 8:212567. 10.7573/dic.212567 30815024PMC6385623

[161] NeelapuSSLockeFLBartlettNLLekakisLJMiklosDBJacobsonCA. Axicabtagene Ciloleucel CAR T-Cell Therapy in Refractory Large B-Cell Lymphoma. New Engl J Med (2017) 377(26):2531–44. 10.1056/NEJMoa1707447 PMC588248529226797

[162] SchusterSJBishopMRTamCSWallerEKBorchmannPMcGuirkJP. Tisagenlecleucel in Adult Relapsed or Refractory Diffuse Large B-Cell Lymphoma. New Engl J Med (2019) 380(1):45–56. 10.1056/NEJMoa1804980 30501490

[163] AbramsonJSPalombaMLGordonLILunningMAWangMLArnasonJE. Pivotal Safety and Efficacy Results From Transcend NHL 001, a Multicenter Phase 1 Study of Lisocabtagene Maraleucel (Liso-Cel) in Relapsed/Refractory (R/R) Large B Cell Lymphomas. Am Soc Hematol Washington DC (2019). 10.1182/blood-2019-127508

[164] LockeFLGhobadiAJacobsonCAMiklosDBLekakisLJOluwoleOO. Long-Term Safety and Activity of Axicabtagene Ciloleucel in Refractory Large B-Cell Lymphoma (ZUMA-1): A Single-Arm, Multicentre, Phase 1–2 Trial. Lancet Oncol (2019) 20(1):31–42. 10.1016/S1470-2045(18)30864-7 30518502PMC6733402

[165] LockeFLNeelapuSSBartlettNLSiddiqiTChavezJCHosingCM. Phase 1 Results of ZUMA-1: A Multicenter Study of KTE-C19 Anti-CD19 Car T Cell Therapy in Refractory Aggressive Lymphoma. Mol Ther (2017) 25(1):285–95. 10.1016/j.ymthe.2016.10.020 PMC536329328129122

[166] JohnsonPCAbramsonJS. Patient Selection for Chimeric Antigen Receptor (CAR) T-Cell Therapy for Aggressive B-Cell Non-Hodgkin Lymphomas. Leuk Lymphoma (2020) 61(11):2561–7. 10.1080/10428194.2020.1786563 32611216

[167] PrasadV. Tisagenlecleucel—The First Approved CAR-T-Cell Therapy: Implications for Payers and Policy Makers. Nat Rev Clin Oncol (2018) 15(1):11–2. 10.1038/nrclinonc.2017.156 28975930

[168] SommermeyerDHudecekMKosasihPLGogishviliTMaloneyDGTurtleCJ. Chimeric Antigen Receptor-Modified T Cells Derived From Defined CD8+ and CD4+ Subsets Confer Superior Antitumor Reactivity *In Vivo* . Leukemia (2016) 30(2):492–500. 10.1038/leu.2015.247 26369987PMC4746098

[169] SavoldoBRamosCALiuEMimsMPKeatingMJCarrumG. CD28 Costimulation Improves Expansion and Persistence of Chimeric Antigen Receptor–Modified T Cells in Lymphoma Patients. J Clin Invest (2011) 121(5):1822–6.10.1172/JCI46110PMC308379521540550

[170] KalosMLevineBLPorterDLKatzSGruppSABaggA. T Cells With Chimeric Antigen Receptors Have Potent Antitumor Effects and can Establish Memory in Patients With Advanced Leukemia. Sci Transl Med (2011) 3(95):95ra73.10.1126/scitranslmed.3002842PMC339309621832238

[171] PorterDLLevineBLKalosMBaggAJuneCH. Chimeric Antigen Receptor–Modified T Cells in Chronic Lymphoid Leukemia. N Engl J Med (2011) 365:725–33.10.1056/NEJMoa1103849PMC338727721830940

[172] KochenderferJNDudleyMEFeldmanSAWilsonWHSpanerDEMaricI. B-Cell Depletion and Remissions of Malignancy Along With Cytokine-Associated Toxicity in a Clinical Trial of Anti-CD19 Chimeric-Antigen-Receptor–Transduced T Cells. Blood Am Soc Hematol (2012) 119(12):2709–20.10.1182/blood-2011-10-384388PMC332745022160384

[173] KochenderferJNRosenbergSA. Treating B-Cell Cancer With T Cells Expressing Anti-CD19 Chimeric Antigen Receptors. Nat Rev Clin Oncol (2013) 10(5):267.2354652010.1038/nrclinonc.2013.46PMC6322669

[174] CruzCRYMicklethwaiteKPSavoldoBRamosCALamSKuS. Infusion of Donor-Derived CD19-Redirected Virus-Specific T Cells for B-Cell Malignancies Relapsed After Allogeneic Stem Cell Transplant: A Phase 1 Study. Blood (2013) 122(17):2965–73.10.1182/blood-2013-06-506741PMC381117124030379

[175] PorterDLHwangW-TFreyNVLaceySFShawPALorenAW. Chimeric Antigen Receptor T Cells Persist and Induce Sustained Remissions in Relapsed Refractory Chronic Lymphocytic Leukemia. Sci Transl Med (2015) 7(303):303ra139.10.1126/scitranslmed.aac5415PMC590906826333935

[176] LeeDWKochenderferJNStetler-StevensonMCuiYKDelbrookCFeldmanSA. T Cells Expressing CD19 Chimeric Antigen Receptors for Acute Lymphoblastic Leukaemia in Children and Young Adults: A Phase 1 Dose-Escalation Trial. Lancet (2015) 385(9967):517–28.10.1016/S0140-6736(14)61403-3PMC706535925319501

[177] BrudnoJNSomervilleRPShiVRoseJJHalversonDCFowlerDH. Allogeneic T Cells That Express an Anti-CD19 Chimeric Antigen Receptor Induce Remissions of B-Cell Malignancies That Progress After Allogeneic Hematopoietic Stem-Cell Transplantation Without Causing Graft-Versus-Host Disease. J Clin Oncol (2016) 34(10):1112.2681152010.1200/JCO.2015.64.5929PMC4872017

[178] TurtleCJHanafiL-ABergerCHudecekMPenderBRobinsonE. Immunotherapy of Non-Hodgkin’s Lymphoma With a Defined Ratio of CD8+ and CD4+ CD19-Specific Chimeric Antigen Receptor–Modified T Cells. Sci Transl Med (2016) 8(355):355ra116.10.1126/scitranslmed.aaf8621PMC504530127605551

[179] WangXPopplewellLLWagnerJRNaranjoABlanchardMSMottMR. Phase 1 Studies of Central Memory–Derived CD19 CAR T–Cell Therapy Following Autologous HSCT in Patients With B-Cell NHL. Blood (2016) 127(24):2980–90.10.1182/blood-2015-12-686725PMC491186227118452

[180] KebriaeiPSinghHHulsMHFigliolaMJBassettROlivaresS. Phase I Trials Using Sleeping Beauty to Generate CD19-Specific CAR T Cells. J Clin Invest (2016) 126(9):3363–76.10.1172/JCI86721PMC500493527482888

[181] TurtleCJHayKAHanafiL-ALiDCherianSChenX. Durable Molecular Remissions in Chronic Lymphocytic Leukemia Treated With CD19-Specific Chimeric Antigen Receptor–Modified T Cells After Failure of Ibrutinib. J Clin Oncol (2017) 35(26):3010.2871524910.1200/JCO.2017.72.8519PMC5590803

[182] EnbladGKarlssonHGammelgårdGWentheJLövgrenTAminiRM. A Phase I/IIa Trial Using CD19-Targeted Third-Generation CAR T Cells for Lymphoma and Leukemia. Clin Cancer Res (2018) 24(24):6185–94.10.1158/1078-0432.CCR-18-042630097433

[183] RamosCARouceRRobertsonCSReynaANaralaNVyasG. *In Vivo* Fate and Activity of Second-Versus Third-Generation CD19-specific CAR-T Cells in B Cell Non-Hodgkin’s Lymphomas. Mol Ther (2018) 26(12):2727–37. 10.1016/j.ymthe.2018.09.009 PMC627748430309819

[184] MajznerRGMackallCL. Tumor Antigen Escape From CAR T-Cell Therapy. Cancer Discov (2018) 8(10):1219–26. 10.1158/2159-8290.CD-18-0442 30135176

[185] RafiqSBrentjensRJ. Tumors Evading CARs—The Chase is on. Nat Med (2018) 24(10):1492–3. 10.1038/s41591-018-0212-6 30297897

[186] ZahELinM-YJensenMCSilva-BenedictAChenYY. Abstract IA12: Combating Antigen Escape With CD19/CD20 Bispecific CAR-T Cell Therapy. AACR (2017). 10.1158/2326-6074.TUMIMM16-IA12

[187] ZhuFShahNXuHSchneiderDOrentasRDropulicB. Closed-System Manufacturing of CD19 and Dual-Targeted CD20/19 Chimeric Antigen Receptor T Cells Using the CliniMACS Prodigy Device at an Academic Medical Center. Cytotherapy (2018) 20(3):394–406. 10.1016/j.jcyt.2017.09.005 29287970

[188] SunLLEllermanDMathieuMHristopoulosMChenXLiY. Anti-CD20/CD3 T Cell–Dependent Bispecific Antibody for the Treatment of B Cell Malignancies. Sci Trans Med (2015) 7(287):287ra70–ra70. 10.1126/scitranslmed.aaa4802 25972002

[189] ChongEASvobodaJDwivedy NastaSLandsburgDJWinchellNNapierE. Sequential Anti-CD19 Directed Chimeric Antigen Receptor Modified T-Cell Therapy (CART19) and PD-1 Blockade With Pembrolizumab in Patients With Relapsed or Refractory B-Cell Non-Hodgkin Lymphomas. Blood (2018) 132(Supplement 1):4198–. 10.1182/blood-2018-99-119502

[190] JacobsonCALockeFLMiklosDBHerreraAFWestinJRLeeJ. End of Phase 1 Results From Zuma-6: Axicabtagene Ciloleucel (Axi-Cel) in Combination With Atezolizumab for the Treatment of Patients With Refractory Diffuse Large B Cell Lymphoma. Biol Blood Marrow Transplant (2019) 25(3):S173. 10.1016/j.bbmt.2018.12.314

[191] SeidelJAOtsukaAKabashimaK. Anti-PD-1 and anti-CTLA-4 Therapies in Cancer: Mechanisms of Action, Efficacy, and Limitations. Front Oncol (2018) 8:86. 10.3389/fonc.2018.00086 29644214PMC5883082

[192] RenJLiuXFangCJiangSJuneCHZhaoY. Multiplex Genome Editing to Generate Universal CAR T Cells Resistant to PD1 Inhibition. Clin Cancer Res (2017) 23(9):2255–66. 10.1158/1078-0432.CCR-16-1300 PMC541340127815355

[193] AzijliKStellooEPetersGJVan den EertweghAJ. New Developments in the Treatment of Metastatic Melanoma: Immune Checkpoint Inhibitors and Targeted Therapies. Anticancer Res (2014) 34(4):1493–505.24692676

[194] DengLLiangHBurnetteBBeckettMDargaTWeichselbaumRR. Irradiation and Anti–PD-L1 Treatment Synergistically Promote Antitumor Immunity in Mice. J Clin Invest (2014) 124(2):687–95. 10.1172/JCI67313 PMC390460124382348

[195] KoneruMO’CearbhaillRPendharkarSSpriggsDRBrentjensRJ. A Phase I Clinical Trial of Adoptive T Cell Therapy Using IL-12 Secreting MUC-16 Ecto Directed Chimeric Antigen Receptors for Recurrent Ovarian Cancer. J Trans Med (2015) 13(1):102. 10.1186/s12967-015-0460-x PMC443863625890361

[196] HoyosVSavoldoBQuintarelliCMahendravadaAZhangMVeraJ. Engineering CD19-Specific T Lymphocytes With Interleukin-15 and a Suicide Gene to Enhance Their Anti-Lymphoma/Leukemia Effects and Safety. Leukemia (2010) 24(6):1160. 10.1038/leu.2010.75 20428207PMC2888148

[197] ChmielewskiMAbkenH. Car T Cells Releasing IL-18 Convert to T-Bethigh FoxO1low Effectors That Exhibit Augmented Activity Against Advanced Solid Tumors. Cell Rep (2017) 21(11):3205–19. 10.1016/j.celrep.2017.11.063 29241547

[198] BatleviCPalombaMParkJMeadESantomassoBRiviereI. Phase I Clinical TRIAL of CD19-TARGETED 19-28Z/4-1BBL “Armored” Car T Cells IN Patients WITH Relapsed OR Refractory NHL and CLL Including RICHTER Transformation. Hematol Oncol (2019) 37:166–7. 10.1002/hon.124_2629

[199] LiuHLeiWZhangCYangCWeiJGuoQ. A Phase I Trial Using CD19 CAR-T Expressing PD-1/CD28 Chimeric Switch-Receptor for Refractory or Relapsed B-cell Lymphoma. Am Soc Clin Oncol (2019) 14:1-5. 10.1200/JCO.2019.37.15_suppl.7557

[200] YoonDHOsbornMJTolarJKimCJ. Incorporation of Immune Checkpoint Blockade Into Chimeric Antigen Receptor T Cells (CAR-Ts): Combination or Built-in CAR-T. Int J Mol Sci (2018) 19(2):340. 10.3390/ijms19020340 PMC585556229364163

[201] SinghNShiJJuneCHRuellaM. Genome-Editing Technologies in Adoptive T Cell Immunotherapy for Cancer. Curr Hematol Malignancy Rep (2017) 12(6):522–9. 10.1007/s11899-017-0417-7 PMC570922429039115

[202] QasimWZhanHSamarasingheSAdamsSAmroliaPStaffordS. Molecular Remission of Infant B-ALL After Infusion of Universal TALEN Gene-Edited CAR T Cells. Sci Trans Med (2017) 9(374). 10.1126/scitranslmed.aaj2013 28123068

[203] JacobsonCAHerreraAFBuddeLEDeAngeloDJHeeryCSteinA. Initial Findings of the Phase 1 Trial of PBCAR0191, A CD19 Targeted Allogeneic CAR-T Cell Therapy. Am Soc Hematol Washington DC (2019) 4107. 10.1182/blood-2019-128203

[204] SotilloEBarrettDMBlackKLBagashevAOldridgeDWuG. Convergence of Acquired Mutations and Alternative Splicing of CD19 Enables Resistance to CART-19 Immunotherapy. Cancer Discovery (2015) 5(12):1282–95. 10.1158/2159-8290.CD-15-1020 PMC467080026516065

[205] GardnerRAFinneyOAnnesleyCBrakkeHSummersCLegerK. Intent-to-Treat Leukemia Remission by CD19 Car T Cells of Defined Formulation and Dose in Children and Young Adults. Blood (2017) 129(25):3322–31. 10.1182/blood-2017-02-769208 PMC548210328408462

[206] GardnerRWuDCherianSFangMHanafiL-AFinneyO. Acquisition of a CD19-Negative Myeloid Phenotype Allows Immune Escape of MLL-Rearranged B-ALL From CD19 Car-T-cell Therapy. Blood (2016) 127(20):2406–10. 10.1182/blood-2015-08-665547 PMC487422126907630

[207] BuddeLEBergerCLinYWangJLinXFrayoSE. Combining a CD20 Chimeric Antigen Receptor and An Inducible Caspase 9 Suicide Switch to Improve the Efficacy and Safety of T Cell Adoptive Immunotherapy for Lymphoma. PLoS One (2013) 8(12):e82742. 10.1371/journal.pone.0082742 24358223PMC3866194

[208] HasoWLeeDWShahNNStetler-StevensonMYuanCMPastanIH. Anti-CD22–chimeric Antigen Receptors Targeting B-Cell Precursor Acute Lymphoblastic Leukemia. Blood (2013) 121(7):1165–74. 10.1182/blood-2012-06-438002 PMC357575923243285

[209] FlavellDJBoehmDAEmeryLMossARamsayAFlavellSU. Therapy of Human B-Cell Lymphoma Bearing Scid Mice is More Effective With Anti-CD19-and Anti-CD38-saporin Immunotoxins Used in Combination Than With Either Immunotoxin Used Alone. Int J Cancer (1995) 62(3):337–44. 10.1002/ijc.2910620318 7543082

[210] DeAngeloDJ. The Use of Novel Monoclonal Antibodies in the Treatment of Acute Lymphoblastic Leukemia. Hematology (2015) 2015(1):400–5. 10.1182/asheducation-2015.1.400 26637749

[211] XuYLiSWangYLiuJMaoXXingH. Induced CD20 Expression on B-cell Malignant Cells Heightened the Cytotoxic Activity of Chimeric Antigen Receptor Engineered T Cells. Hum Gene Ther (2019) 30(4):497–510. 10.1089/hum.2018.119 30381966

[212] SteidlCGascoyneRD. The Molecular Pathogenesis of Primary Mediastinal Large B-Cell Lymphoma. Blood (2011) 118(10):2659–69. The Journal of the American Society of Hematology. 10.1182/blood-2011-05-326538 21700770

[213] BossardCDobayMPParrensMLamantLMissiagliaEHaiounC. Immunohistochemistry as a Valuable Tool to Assess CD30 Expression in Peripheral T-Cell Lymphomas: High Correlation With mRNA Levels. Blood (2014) 124(19):2983–6. The Journal of the American Society of Hematology. 10.1182/blood-2014-07-584953 25224410

[214] SabattiniEPizziMTabanelliVBaldinPSacchettiCSAgostinelliC. CD30 Expression in Peripheral T-Cell Lymphomas. Haematologica (2013) 98(8):e81–e2. 10.3324/haematol.2013.084913 PMC372988623716537

[215] BergerGKGeeKVotrubaCMcBrideAAnwerF. Potential Application and Prevalence of the CD30 (Ki-1) Antigen Among Solid Tumors: A Focus Review of the Literature. Crit Rev Oncol/Hematol (2017) 113:8–17. 10.1016/j.critrevonc.2017.02.021 28427526

[216] BonthapallyVWuEMacalaladAYangHShonukanOLiuY. Brentuximab Vedotin in Relapsed/Refractory Hodgkin Lymphoma Post-Autologous Transplant: Meta-Analysis Versus Historical Data. Curr Med Res Opin (2015) 31(5):993–1001. 10.1185/03007995.2015.1030378 25772232

[217] ThurberGMSchmidtMMWittrupKD. Antibody Tumor Penetration: Transport Opposed by Systemic and Antigen-Mediated Clearance. Adv Drug Deliv Rev (2008) 60(12):1421–34. 10.1016/j.addr.2008.04.012 PMC282030718541331

[218] SavoldoBRooneyCMDi StasiAAbkenHHombachAFosterAE. Epstein Barr Virus–Specific Cytotoxic T Lymphocytes Expressing the Anti-CD30ζ Artificial Chimeric T-cell Receptor for Immunotherapy of Hodgkin Disease. Blood (2007) 110(7):2620–30. The Journal of the American Society of Hematology. 10.1182/blood-2006-11-059139 PMC198894417507664

[219] Di StasiADe AngelisBRooneyCMZhangLMahendravadaAFosterAE. T Lymphocytes Coexpressing CCR4 and a Chimeric Antigen Receptor Targeting CD30 Have Improved Homing and Antitumor Activity in a Hodgkin Tumor Model. Blood (2009) 113(25):6392–402. The Journal of the American Society of Hematology. 10.1182/blood-2009-03-209650 PMC271093219377047

[220] WangC-MWuZ-QWangYGuoY-LDaiH-RWangX-H. Autologous T Cells Expressing CD30 Chimeric Antigen Receptors for Relapsed or Refractory Hodgkin Lymphoma: An Open-Label Phase I Trial. Clin Cancer Res (2017) 23(5):1156–66. 10.1158/1078-0432.CCR-16-1365 27582488

[221] RamosCABallardBZhangHDakhovaOGeeAPMeiZ. Clinical and Immunological Responses After CD30-specific Chimeric Antigen Receptor–Redirected Lymphocytes. J Clin Invest (2017) 127(9):3462–71. 10.1172/JCI94306 PMC566957328805662

[222] GuercioMOrlandoDDi CeccaSSinibaldiMBoffaICarusoS. Cd28. OX40 Co-Stimulatory Combination is Associated With Long *In Vivo* Persistence and High Activity of CAR. CD30 T-cells Haematol (2020) 166:987. 10.3324/haematol.2019.231183 PMC801815832381575

[223] BarrenaSAlmeidaJYuntaMLópezAFernandez-MosteirinNGiraltM. Aberrant Expression of Tetraspanin Molecules in B-Cell Chronic Lymphoproliferative Disorders and Its Correlation With Normal B-Cell Maturation. Leukemia (2005) 19(8):1376–83. 10.1038/sj.leu.2403822 15931266

[224] De WindeCMVeenbergenSYoungKHXu-MonetteZYX-xWXiaY. Tetraspanin CD37 Protects Against the Development of B Cell Lymphoma. J Clin Invest (2016) 126(2):653–66. 10.1172/JCI81041 PMC473117726784544

[225] de WindeCMElfrinkSvan SprielAB. Novel Insights Into Membrane Targeting of B Cell Lymphoma. Trends Cancer (2017) 3(6):442–53. 10.1016/j.trecan.2017.04.006 28718418

[226] BertoniFStathisA. Staining the Target: CD37 Expression in Lymphomas. Blood Am Soc Hematol (2016) 128(26):3022–3. 10.1182/blood-2016-11-748137 28034866

[227] ScarfòIOrmhøjMFrigaultMJCastanoAPLorreySBouffardAA. Anti-CD37 Chimeric Antigen Receptor T Cells Are Active Against B-and T-Cell Lymphomas. Blood (2018) 132(14):1495–506. 10.1182/blood-2018-04-842708 PMC617256430089630

[228] RuellaMXuJBarrettDMFraiettaJAReichTJAmbroseDE. Induction of Resistance to Chimeric Antigen Receptor T Cell Therapy by Transduction of a Single Leukemic B Cell. Nat Med (2018) 24(10):1499–503. 10.1038/s41591-018-0201-9 PMC651198830275568

[229] KöksalHDillardPJosefssonSEMaggadottirSMPollmannSFåneA. Preclinical Development of CD37CAR T-Cell Therapy for Treatment of B-cell Lymphoma. Blood Adv (2019) 3(8):1230–43. 10.1182/bloodadvances.2018029678 PMC648236030979721

[230] VooijsWSchuurmanHBastEDe GastG. Evaluation of CD38 as Target for Immunotherapy in Multiple Myeloma. Blood (1995) 15:2282–4. 10.1182/blood.V85.8.2282.bloodjournal8582282 7718903

[231] MehtaKOcanasLMalavasiFMarksJWRosenblumMG. Retinoic Acid-Induced CD38 Antigen as a Target for Immunotoxin-Mediated Killing of Leukemia Cells. Mol Cancer Ther (2004) 3(3):345–52.15026555

[232] PengK-WDonovanKASchneiderUCattaneoRLustJARussellSJ. Oncolytic Measles Viruses Displaying a Single-Chain Antibody Against CD38, A Myeloma Cell Marker. Blood (2003) 101(7):2557–62. The Journal of the American Society of Hematology. 10.1182/blood-2002-07-2195 12433686

[233] GoldmacherVSBourretLALevineBARasmussenRAPourshadiMLambertJM. Anti-CD38-Blocked Ricin: An Immunotoxin for the Treatment of Multiple Myeloma. Blood (1994) 184:3017–25. 10.1182/blood.V84.9.3017.3017 7524764

[234] MiharaKYanagiharaKTakigahiraMKitanakaAImaiCBhattacharyyaJ. Synergistic and Persistent Effect of T-Cell Immunotherapy With Anti-CD19 or Anti-CD38 Chimeric Receptor in Conjunction With Rituximab on B-Cell Non-Hodgkin Lymphoma. Br J Haematol (2010) 151(1):37–46. 10.1111/j.1365-2141.2010.08297.x 20678160

[235] KallamAVoseJM. Recent Advances in CAR-T Cell Therapy for Non-Hodgkin Lymphoma. Clin Lymphoma Myeloma Leuk (2019) 19(12):751–7. 10.1016/j.clml.2019.09.598 31648957

[236] SalterAIIveyRGKennedyJJVoilletVRajanAAldermanEJ. Phosphoproteomic Analysis of Chimeric Antigen Receptor Signaling Reveals Kinetic and Quantitative Differences That Affect Cell Function. Sci Signaling (2018) 11(544):eaat6753. 10.1126/scisignal.aat6753 PMC618642430131370

[237] MaudeSLFreyNShawPAAplencRBarrettDMBuninNJ. Chimeric Antigen Receptor T Cells for Sustained Remissions in Leukemia. New Engl J Med (2014) 371(16):1507–17. 10.1056/NEJMoa1407222 PMC426753125317870

[238] BrudnoJNKochenderferJN. Recent Advances in CAR T-Cell Toxicity: Mechanisms, Manifestations and Management. Blood Rev (2019) 34:45–55. 10.1016/j.blre.2018.11.002 30528964PMC6628697

[239] NeelapuSSTummalaSKebriaeiPWierdaWGutierrezCLockeFL. Chimeric Antigen Receptor T-Cell Therapy—Assessment and Management of Toxicities. Nat Rev Clin Oncol (2018) 15(1):47. 10.1038/nrclinonc.2017.148 28925994PMC6733403

[240] LeeDWGardnerRPorterDLLouisCUAhmedNJensenM. Current Concepts in the Diagnosis and Management of Cytokine Release Syndrome. Blood (2014) 124(2):188–95. 10.1182/blood-2014-05-552729 PMC409368024876563

[241] FreyN. Cytokine Release Syndrome: Who is at Risk and How to Treat. Best Pract Res Clin Haematol (2017) 30(4):336–40. 10.1016/j.beha.2017.09.002 29156206

[242] DavilaMLRiviereIWangXBartidoSParkJCurranK. Efficacy and Toxicity Management of 19-28z Car T Cell Therapy in B Cell Acute Lymphoblastic Leukemia. Sci Trans Med (2014) 6(224):224ra25–ra25. 10.1126/scitranslmed.3008226 PMC468494924553386

[243] PishkoANastaSD. The Role of Novel Immunotherapies in non-Hodgkin Lymphoma. Trans Cancer Res (2017) 6(1):93. 10.21037/tcr.2017.01.08 PMC561237128955654

[244] LeRQLiLYuanWShordSSNieLHabtemariamBA. FDA Approval Summary: Tocilizumab for Treatment of Chimeric Antigen Receptor T Cell-Induced Severe or Life-Threatening Cytokine Release Syndrome. Oncol (2018) 23(8):943. 10.1634/theoncologist.2018-0028 PMC615617329622697

[245] RiceJNagelSRandallJHinsonHE. Chimeric Antigen Receptor T Cell-Related Neurotoxicity: Mechanisms, Clinical Presentation, and Approach to Treatment. Curr Treat Options Neurol (2019) 21(8):40. 10.1007/s11940-019-0580-3 31327064

[246] JacksonSWheatleyT. Chimeric Antigen Receptor T-Cell Emergencies: Inpatient Administration, Assessment, and Management. Semin Oncol Nurs (2021) 151134. 10.1016/j.soncn.2021.151134 33795179

[247] GustJTaraseviciuteATurtleCJ. Neurotoxicity Associated With CD19-targeted CAR-T Cell Therapies. CNS Drugs (2018) 32(12):1091–101. 10.1007/s40263-018-0582-9 PMC729511530387077

[248] BrudnoJNKochenderferJN. Toxicities of Chimeric Antigen Receptor T Cells: Recognition and Management. Blood (2016) 127(26):3321–30. 10.1182/blood-2016-04-703751 PMC492992427207799

[249] CrumpMKuruvillaJCoubanSMacDonaldDAKukretiVKouroukisCT. Randomized Comparison of Gemcitabine, Dexamethasone, and Cisplatin Versus Dexamethasone, Cytarabine, and Cisplatin Chemotherapy Before Autologous Stem-Cell Transplantation for Relapsed and Refractory Aggressive Lymphomas: NCIC-CTG Ly. J Clin Oncol (2014) 12:3490-6. 10.1200/JCO.2013.53.9593 25267740

[250] Van ImhoffGWMcMillanAMatasarMJRadfordJArdeshnaKMKuliczkowskiK. Ofatumumab Versus Rituximab Salvage Chemoimmunotherapy in Relapsed or Refractory Diffuse Large B-Cell Lymphoma: The ORCHARRD Study. J Clin Oncol (2017) 35(5):544–51. 10.1200/JCO.2016.69.0198 28029326

[251] KuramitsuSOhnoMOhkaFShiinaSYamamichiAKatoA. Lenalidomide Enhances the Function of Chimeric Antigen Receptor T Cells Against the Epidermal Growth Factor Receptor Variant III by Enhancing Immune Synapses. Cancer Gene Ther (2015) 22(10):487–95. 10.1038/cgt.2015.47 26450624

[252] ZhengWCarolEAlliRBashamJHAbdelsamedHAPalmerLE. PI3K Orchestration of the *In Vivo* Persistence of Chimeric Antigen Receptor-Modified T Cells. Leukemia (2018) 32(5):1157–67. 10.1038/s41375-017-0008-6 PMC594319129479065

[253] RuellaMKenderianSSShestovaOFraiettaJAQayyumSZhangQ. The Addition of the BTK Inhibitor Ibrutinib to anti-CD19 Chimeric Antigen Receptor T Cells (CART19) Improves Responses Against Mantle Cell Lymphoma. Clin Cancer Res (2016) 22(11):2684–96. 10.1158/1078-0432.CCR-15-1527 26819453

[254] CherkasskyLMorelloAVillena-VargasJFengYDimitrovDSJonesDR. Human CAR T Cells With Cell-Intrinsic PD-1 Checkpoint Blockade Resist Tumor-Mediated Inhibition. J Clin Invest (2016) 126(8):3130–44. 10.1172/JCI83092 PMC496632827454297

[255] FryTJShahNNOrentasRJStetler-StevensonMYuanCMRamakrishnaS. CD22-Targeted CAR T Cells Induce Remission in B-ALL That is Naive or Resistant to CD19-targeted CAR Immunotherapy. Nat Med (2018) 24(1):20. 10.1038/nm.4441 29155426PMC5774642

[256] EyquemJMansilla-SotoJGiavridisTvan der StegenSJHamiehMCunananKM. Targeting a CAR to the TRAC Locus With CRISPR/Cas9 Enhances Tumour Rejection. Nature (2017) 543(7643):113–7. 10.1038/nature21405 PMC555861428225754

[257] KoneruMPurdonTJSpriggsDKoneruSBrentjensRJ. Il-12 Secreting Tumor-Targeted Chimeric Antigen Receptor T Cells Eradicate Ovarian Tumors *In Vivo* . Oncoimmunology (2015) 4(3):e994446. 10.4161/2162402X.2014.994446 25949921PMC4404840

[258] AvanziMPYekuOLiXWijewarnasuriyaDPvan LeeuwenDGCheungK. Engineered Tumor-Targeted T Cells Mediate Enhanced Anti-Tumor Efficacy Both Directly and Through Activation of the Endogenous Immune System. Cell Rep (2018) 23(7):2130–41. 10.1016/j.celrep.2018.04.051 PMC598628629768210

[259] PoirotLPhilipBSchiffer-ManniouiCLe ClerreDChion-SotinelIDerniameS. Multiplex Genome-Edited T-Cell Manufacturing Platform for “Off-the-Shelf” Adoptive T-Cell Immunotherapies. Cancer Res (2015) 75(18):3853–64. 10.1158/0008-5472.CAN-14-3321 26183927

